RETRACTED

# Picture Fuzzy Einstein Hybrid-Weighted Aggregation Operator and Its Application to Multicriteria Group Decision Making

**DOI:** 10.1155/2022/6925670

**Published:** 2022-05-14

**Authors:** Guo Cao

**Affiliations:** School of Economics and Management, Changzhou Institute of Technology, Changzhou 213032, China

## Abstract

As an extension of intuitionistic fuzzy sets (IFSs), picture fuzzy sets (PFSs) can better model and represent the hesitancy and uncertainty of decision makers' preference information. In this study, we propose a multicriteria group decision making (MCGMD) method based on picture fuzzy sets. We first define some basic picture Einstein operations with closed properties among PFSs on the basis of the Einstein t-norms and t-conorms. Then, utilizing the hybrid-weighted operator and the developed picture Einstein operations laws, we put forward a picture fuzzy Einstein hybrid-weighted aggregation operator for aggregating PFSs and discuss its several important properties. Furthermore, we present a new MCGMD method based on the proposed picture fuzzy Einstein hybrid-weighted aggregation operator. Finally, an example is conducted to validate the effectiveness of the proposed MCGMD method.

## 1. Introduction

Multicriteria group decision making (MCGDM) is one of the most important human activities [1–6]. Due to the complexity and vagueness of information in group decision making, however, it is usually difficult for decision makers to evaluate the alternatives by crisp numerical values [7, 8]. In some occasions, it can be more reasonable to give uncertain or fuzzy evaluation information represented by fuzzy numbers [9, 10], intuitionistic fuzzy sets (IFS) [11–15], neutrosophic set (NS) [16–18], Pythagorean fuzzy sets [19, 20], Fermatean fuzzy sets [21, 22], hesitant fuzzy sets [23–25], and so on. Based on the concept of fuzzy sets (FSs), Atanassov [26] first introduced the concept of IFS, which is an extension of Zadeh's FSs. Different from FSs, it does not require that the sum of the degrees of membership and non-membership of an element to be equal to one. IFSs have been successfully applied to multicriteria group decision making. However, there are some scenarios that cannot be represented by IFSs in some real-life group decision-making problems, such as the option of hesitation or remaining neutral. To overcome this drawback, Smarandache [27] proposed the concept of the NS, which has the degrees of truth, falsity, and indeterminacy, respectively. Considering that it is difficult to utilize NSs to solve real-life scientific and engineering problems, Zhang and Sunderraman [28] proposed the concept of the single-valued neutrosophic set (SVNS). In this paper, Boran and Akay [11] also developed some set-theoretic operators and discussed their various properties. Compared with NS, it is assumed in a SVNS that each type of membership degree can take its values in the interval [0, 1], and the sum of its truth-membership degree, indeterminacy-membership degree, and false-membership degree is less than or equal to 3. This hypothesis implies that its three types of membership degrees do not satisfy probabilistic independence. This non-restriction leads to dialetheist and paraconsistent information in real-life decision-making problems represented as SVNSs. In order to overcome these drawbacks of IFSs and NSs, Cuong and Kreinovich [29] proposed the concept of the picture fuzzy set (PFS) to address a fact such that human opinions involve several types of answers such as yes, abstain, no, or refusal and so on. The PFS is characterized by a positive membership function, a negative membership function, and a neutral membership function, and the sum of its three membership degrees is less than or equal to 1. Different from NS, there is a restriction on the sum of the three types of membership degrees in PFS, which implies that they are dependent on each other.

RETRACTED

The PFS is an extension of FS and IFS [30]. The core of PFS is its picture fuzzy value (PFV), which is composed of the degree of positive, negative, and neutral memberships. Similar to an intuitionistic fuzzy value (IFV) and NS, PFV is also a very effective tool to express inherent uncertainty or imprecision of decision makers' preference information in human decision-making processes. Recently, PFS has been successfully applied to a lot of areas. For example, Zhang et al. [23] introduced the concept of generalized picture distance measure and applied it to pattern recognition. Based on the correlation measure of Atanassov' s IFSs, Singh [31] also proposed the concept of correlation for PFSs to solve bidirectional approximate reasoning systems problems. By combining picture composite cardinality with PSO, Thong and Son [32] proposed a novel automatic picture fuzzy clustering method for pattern recognition and knowledge discovery.

In the course of MCGMD with IFS, hesitant fuzzy set, and NS, the aggregation operators play a very important role [33]. Many scholars have introduced various aggregation operators for IFS, hesitant fuzzy set, and NS, such as intuitionistic fuzzy aggregation operators [34], hesitant fuzzy aggregation operators [35], interval-valued intuitionistic fuzzy aggregation operators [36], the neutrosophic fuzzy aggregation operators [37, 38] picture fuzzy aggregation operators [39–41], and so on. Note that most of the abovementioned aggregation operators were developed based on the triangular t-norm and t-conorm for the following reasons. For IFSs, they only involve membership degree and non-membership degree such that their sum is less than or equal to 1. Thus, triangular t-norms and t-conorms are appropriate in developing the intuitionistic fuzzy aggregation operators. As for SVNS, the sum of its truth-membership degree, indeterminacy-membership degree, and false-membership degree is less than or equal to 3. Hence, triangular t-norm or t-conorm could be directly used to synthesize separate NSs into a collective one. Although NSs and PFSs both have three kinds of membership functions, their property regarding membership functions is different from each other. This means that the neutrosophic aggregation operators cannot be directly used to aggregate PFSs. For example, let *A*_1_ = (0, 1, 0) and *A*_2_ = (0, 0, 1) be two PFSs. According to the generalized union of SVNSs defined in [32], we have *A*_1_ ⊗ *A*_2_**=**(0,1,1). This result does not satisfy the condition required by PFV that the sum of its membership degrees is less than or equal to 1.

RETRACTED

The algebraic product and algebraic sum are usually used to develop the aggregation operators for FSs [42], IFSs [43], and NSs [44, 45]. There are also other operational rules that can be used in this respect. For example, Einstein t-norms and Einstein t-conorms are two typical classes of strict Archimedean t-norms and t-conorms for aggregating a collection of intuitionistic fuzzy values (IFVs). In this direction, Wang and Liu [46] introduced the intuitionistic fuzzy aggregation operators by using Einstein operations and developed some intuitionistic fuzzy Einstein aggregation operators. Wang and Liu [47] furthermore developed some new intuitionistic fuzzy geometric Einstein aggregation operators. Recently, Einstein t-norms and t-conorms have also been used to aggregate neutrosophic sets and neutrosophic hesitant fuzzy sets, such as the neutrosophic number-generalized weighted power averaging operator [48], and the interval neutrosophic hesitant fuzzy generalized weighted average operator [49]. Among these Einstein aggregation operators; however, some only weight the fuzzy values and others only weight the ordered positions of the fuzzy values similar to the ordered weighted averaging (OWA) operator. To overcome this drawback, Zhao and Wei [50] proposed some new intuitionistic fuzzy Einstein hybrid aggregation operators to aggregate IFVs by combining the weighted average and the OWA operator, such as the intuitionistic fuzzy Einstein hybrid averaging operator and intuitionistic fuzzy Einstein hybrid geometric averaging operator. They weight not only the given arguments but also their ordered positions. However, all of them do not satisfy the desired properties for aggregation operators such as boundedness and idempotency. Recently, some new picture fuzzy aggregation operators are proposed to apply to multicriteria group decision making, such as picture fuzzy Einstein aggregation operators, picture fuzzy-weighted average operators, picture fuzzy-weighted geometric operators, and picture fuzzy Dombi aggregation operators, etc. Although the approaches of MCGMD based on fuzzy aggregation operators have been widely investigated, the existing aggregation operators have the following shortcomings in the aggregation process:

1. IFS cannot well describe inconsistent, hesitation, and indeterminate information, and it does not address the influence of hesitation or neutral fuzzy information on aggregating results in the aggregation process. Thus, the MCGDM method based on intuitionistic fuzzy aggregation operators has the drawback that it may lead to unreasonable decision-making in some situations.
2. The neutrosophic fuzzy hybrid aggregation operators have no occasion to prove that they must satisfy the probabilistic property of the tri-membership function. In some situations, if hybrid aggregation operators are applied in specific NSs, such as intuitionistic neutrosophic sets (INSs) whose sum of tri-membership degrees is required to be less than to 1, the aggregating set is no longer an INS. For example, let *A* = (0, 0.9, 0) and *B* = (0, 0, 0.9) be two INSs. According to the inner product operation defined in [51], we obtain *A*⊗*B* = (0, 0.9, 0.9), which implies that the aggregating set is no longer an INS. Thus, it is important to develop new neutrosophic fuzzy hybrid aggregation operators which are suitable to all types of NSs.
3. Picture fuzzy multicriteria group decision making problem will be a new direction for group decision making. However, the existing Einstein aggregation operators for NSs cannot be directly applied in picture fuzzy environments. Moreover, most of these existing neutrosophic Einstein hybrid aggregation operators do not satisfy some properties such as boundedness and idempotency for picture fuzzy sets. It is, therefore, necessary to extend the existing neutrosophic Einstein aggregation operators to picture fuzzy environments and to propose some new Einstein aggregation operators for aggregating picture fuzzy information. To the best of our knowledge, however, there are no researches on the combination between the PFSs and MCMGD, and how to aggregate PFSs is still an open problem, which is the focus of this paper.

RETRACTED

According to the above discussions, we can see that it is better to consider both the operations rules and aggregation operators for PFSs. The main contribution of this work is as follows:

1. We present some picture fuzzy Einstein operational laws based on Einstein t-norms and t-conorms and discuss their desirable properties.
2. We introduce a new picture fuzzy Einstein hybrid-weighted aggregation (*PFIEHWA*) operator to aggregate PFSs. Based on the proposed aggregation operator, we develop a MAGDM method and validate its effectiveness.

The remaining sections of this paper is organized as follows. In the next section, we introduce some basic concepts related to PFSs and Einstein operations. In Section 3, by extending the Einstein t-conorm and t-norm, we develop several new Einstein operations laws for PFVs, such as generalized intersection and union, and then we discuss their desirable properties. In Section 4, we develop a picture fuzzy Einstein hybrid aggregation operator for PFVs and discuss their desirable properties. In Section 5, we apply the picture fuzzy Einstein hybrid-weighted aggregation operator to a MCGMD problem. Some numerical examples are given to verify the developed approach and to demonstrate its practicality and effectiveness.  Section 6 concludes the paper.

## 2. Preliminaries

In this section, we present some basic definitions and results for IFS and PFS.

**Definition 1 (18).**

An intuitionistic fuzzy set (IFS) *A* in a finite set *X* can be written as follows:

(1) $$\begin{array}{c} \mathrm{A=}\left\{<x,\mu_{A}\left(x\right),\nu_{A}\left(x\right),>,x\in X\right\}, \end{array}$$

where *μ*_*A*_(*x*) and *ν*_*A*_(*x*) : *X*⟶[0,1] are, respectively, the degrees of membership and non-membership such that 0 ≤ *μ*_*A*_(*x*) + *ν*_*A*_(*x*) ≤ 1. For each IFS *A* in a finite set *X*, the hesitancy degree of an IFS *A* can be expressed as *π*_*A*_(*x*) = 1 − *μ*_*A*_(*x*) − *ν*_*A*_(*x*), *x* ∈ *X*. Also, we have 0 ≤ *π*_*A*_(*x*) ≤ 1, for all *x* ∈ *X*.

**Definition 2 (5).**

A picture fuzzy set (PFS) *A* in a finite set *X* is defined as follows:

(2) $$\begin{array}{c} \mathrm{A=}\left\{<x,\mu_{A}\left(x\right),\nu_{A}\left(x\right),\gamma_{A}\left(x\right)>,x\in X\right\}, \end{array}$$

where *μ*_*A*_(*x*), *ν*_*A*_(*x*), and *γ*_*A*_(*x*) represent the positive-membership function, negative-membership function, and neutral-membership function of *x* to set *A*, respectively. For each element *x* in *X*, we have *μ*_*A*_(*x*), *ν*_*A*_(*x*), *γ*_*A*_(*x*)⟶[0,1] and 0 ≤ *μ*_*A*_(*x*) + *ν*_*A*_(*x*) + *γ*_*A*_(*x*) ≤ 1.

Similar to the IFS, *π*_*A*_(*x*)=1 − (*μ*_*A*_(*x*)+*ν*_*A*_(*x*)+*γ*_*A*_(*x*)) could be called the refusal-membership degree of *x* in *A*. For convenience, we can use *x=*(*μ*_*A*_, *ν*_*A*_, *γ*_*A*_) to represent an element in PFSs.

RETRACTED

**Definition 3 (52).**

Let *α* = (*μ*_*α*_, *ν*_*α*_, *γ*_*α*_) be a PFV, and its score function *S*_*α*_ and accuracy function *V*_*α*_ are, respectively, defined as follows:

(3) $$\begin{array}{c} S_{\alpha }=\mu_{\alpha }-\nu_{\alpha },\\ V_{\alpha }=\mu_{\alpha }+\nu_{\alpha }+\gamma_{\alpha }. \end{array}$$

**Theorem 1 (53).**

Let *α*_1_ and *α*_2_ be two PFVs, and the ranking rules between them are given as follows:

(1) If *S*(*α*_1_) > *S*(*α*_2_), then *α*_1_ > *α*_2_
(2) If *S*(*α*_1_) < *S*(*α*_2_), then *α*_1_ < *α*_2_
(3) If *S*(*α*_1_)=*S*(*α*_2_), then
  1. If *V*(*α*_1_)=*V*(*α*_2_), then *α*_1_=*α*_2_
  2. If *V*(*α*_1_) > *V*(*α*_2_), then *α*_1_ > *α*_2_

**Definition 4 .**

Let *PFS(X)* denote the set of all the PFSs in a finite set *X*. Given any two PFSs *A* and *B*, their inclusion, union, intersection, and complement are defined as follows:

1. *A*⊆*Bif*∀*x* ∈ *X*, *μ*_*A*_(*x*) ≤ *μ*_*B*_(*x*), *ν*_*A*_(*x*) ≥ *ν*_*B*_(*x*), *γ*_*A*_(*x*) ≥ *γ*_*B*_(*x*)
2. *A*=*Bif*∀*x* ∈ *X*, *A*⊆*B* and *A*⊇*B*
3. *A* ∪ *B*={*x*, (max(*μ*_*A*_(*x*), *μ*_*B*_(*x*)), min(*ν*_*A*_(*x*), *ν*_*B*_(*x*)), min(*γ*_*A*_(*x*), *γ*_*B*_(*x*)))}
4. *A*∩*B*={*x*, (min(*μ*_*A*_(*x*), *μ*_*B*_(*x*)), max(*ν*_*A*_(*x*), *ν*_*B*_(*x*)), min(*γ*_*A*_(*x*), *γ*_*B*_(*x*)))}
5. coA=*A*^*c*^={<*x*, *ν*_*A*_(*x*), *μ*_*A*_(*x*), *γ*_*A*_(*x*) > , *x* ∈ *X*}

## 3. Picture Fuzzy Einstein Operational Laws

Triangular t-norms and t-conorms play a prominent role for aggregating fuzzy sets in group decision making. Roychowdhury and Wang [53] gave some definitions and conditions for the triangular t-norm and t-conorm, which satisfy the requirements of both conjunction and disjunction operators. The set-theoretical properties of these operators for IFSs generally hold for IFS. In the following section, triangular t-norms and t-conorms are defined as given below:

**Definition 5 (54).**

A function T: [0, 1]^2^⟶ [0, 1] is called a t-norm if it satisfies the following four conditions:

1. *T*(1, *x*)=*x*, ∀*x* ∈ [0,1]
2. *T*(*x*, *y*)=*T*(*y*, *x*), ∀(*x*, *y*) ∈ [0,1]^2^
3. *T*(*x*, *T*(*y*, *z*))=*T*(*T*(*x*, *y*), *z*))∀ (*x*, *y*, *z*) ∈ [0,1]^3^
4. If *x* ≤ *x*′ and *y* ≤  y′, then *T*(*x*, *y*) ≤ *T*(*x*′, *y*′), ∀(*x*, *y*, *x*′, *y*′) ∈ [0,1]^4^

**Definition 6 (54).**

A function S: [0, 1]^2^⟶ [0, 1] is called as a t-conorm if it satisfies the following four conditions:

1. *S*(*x*, 0)=0, ∀*x* ∈ [0,1]
2. *S*(*x*, *y*)=*S*(*y*, *x*), ∀(*x*, *y*) ∈ [0,1]^2^
3. *S*(*x*, *S*(*y*, *z*)) = *S*(*S*(*x*, *y*), *z*), ∀(*x*, *y*, *z*) ∈ [0, 1]^3^
4. If *x* ≤ *x*′ and *y* ≤  y′, then *S*(*x*, *y*) ≤ *S*(*x*′, *y*′), ∀(*x*, *y*, *x*′, *y*′) ∈ [0,1]^4^

Analogous operators on fuzzy sets have also been defined on IFSs. For example, the inclusion of two IFSs can be defined by using the algebraic t-norm for their membership degrees and the algebraic t-conorm for their non-membership degrees, and their inclusion is still an intuitionistic fuzzy set. This is because they are related by the De Morgan duality, *i.e.*, the t-conorm S can be defined as *S*(*x*, *y*)=1 − *T*(1 − *x*, 1 − *y*), ∀(*x*, *y*) ∈ [0,1]^2^. In recent years, triangular t-norms and t-conorms have also been used to define the operation laws for NSs [55]. Although PFV is a generalization of NS, their properties regarding membership functions are different from each other. This means that the operational laws for NSs cannot be directly used to aggregate PFVs. For example, with algebraic t-norm and t-conorm, the union operation for NSs is defined as *A* ∪ *B*=(*T*_1_*T*_2_, *I*_1_+*I*_2_ − *I*_1_*I*_2_, *F*_1_+*F*_2_ − *F*_1_*F*_2_). However, if they are extended to PFVs, there are some limitations. For instance, let *A*=(*x*, 1,0,0) and *B*=(*x*, 0,1,0) be two PFVs. It is clear that *B* is the smallest one among all PFVs. According to the generalized union operation mentioned above, we obtain *A*∪_*S*,*T*_*B*=(*x*, 0,1,0). This means that the aggregating result is also the smallest PFV. Therefore, the operation “union” cannot be accepted because it is against our intuition. Furthermore, let *C*=(*x*, 0,1,0) and *D*=(*x*, 0,0,1) be two PFVs, we also have *μ*_*C*∪*D*_+*ν*_*C*∪*D*_+*γ*_*C*∪*D*_=2 > 1, and this result does not satisfy the condition required by a PFV that the sum of its membership degrees is less than or equal to 1. Thus, it is important to develop the operational rules for PFVs. Motivated by Definition 5 and Definition 6, we first propose a generalized intersection and union for PFVs based on triangular t-norm and t-conorm.

RETRACTED

**Definition 7 .**

Let *α*_*j*_ = (*μ*_*j*_, *ν*_*j*_, *γ*_*j*_), (*j* = 1,2) be two PFVs. The generalized intersection and union between *α*_1_and*α*_2_ are, respectively, defined as follows:

(4) $$\begin{array}{c} \alpha_{1}{⊕}_{S,T}\alpha_{2}=\left(S\left(\mu_{1},\mu_{2}\right),T\left(\nu_{1},\nu_{2}\right),T\left(\gamma_{1},\gamma_{2}\right)\right),\\ \alpha_{1}{⊗}_{S,T}\alpha_{2}=\left(T\left(\mu_{1},\mu_{2}\right),S\left(\nu_{1},\nu_{2}\right),T\left(\gamma_{1},\gamma_{2}\right)\right). \end{array}$$

There are lots of operators based on the algebraic operation which are one of the general concepts of the t-norms and t-conorms. Einstein operation, including the Einstein product and the Einstein sum, also belongs to the t-norms and t-conorms families. Let additive generator*N*(*x*) = 1 − *x*, then Einstein product ⊗_*ε*_ and Einstein sum ⊕_*ε*_ are defined as follows [36]:

1. *α*⊗_*ε*_*β* = *αβ*/(1 + (1 − *α*)(1 − *β*)), ∀(*α*, *β*) ∈ [0,1]
2. *α*⊕_*ε*_*β* = (*α* + *β*)/(1 + *αβ*), ∀(*α*, *β*) ∈ [0,1]

With the abovementioned analysis, the operations laws for PFVs based on Einstein t-norms and t-conorms can be defined as follows:

**Definition 8 .**

Let*α* = (*μ*, *ν*, *γ*) and *α*_*j*_ = (*μ*_*j*_, *ν*_*j*_, *γ*_*j*_), *j* *=* 1, 2, be PFVs, and *λ* is a positive real number. Let additive generator *N*(*x*) = 1 − *x*, then we have the following operations laws:

(5) $$\begin{array}{c} \alpha_{1}{⊕}_{\varepsilon }\alpha_{2}=\left(\frac{\mu_{1}+\mu_{2}}{1+\mu_{1}\mu_{2}},\frac{\nu_{1}\nu_{2}}{1+\left(1-\nu_{1}\right)\left(1-\nu_{2}\right)},\frac{\gamma_{1}\gamma_{2}}{1+\left(1-\gamma_{1}\right)\left(1-\gamma_{2}\right)}\right), \end{array}$$

(6) $$\begin{array}{c} \alpha_{1}{⊗}_{\varepsilon }\alpha_{2}=\left(\frac{u_{1}u_{2}}{1+\left(1-u_{1}\right)\left(1-u_{2}\right)},\frac{\nu_{1}+\nu_{2}}{1+\nu_{1}\nu_{2}},\frac{\gamma_{1}\gamma_{2}}{1+\left(1-\gamma_{1}\right)\left(1-\gamma_{2}\right)}\right), \end{array}$$

(7) $$\begin{array}{c} \lambda \cdot_{\varepsilon }\alpha =\left(\frac{{\left(1+\mu \right)}^{\lambda }-{\left(1-\mu \right)}^{\lambda }}{{\left(1+\mu \right)}^{\lambda }+{\left(1-\mu \right)}^{\lambda }},\frac{2\nu^{\lambda }}{{\left(2-\nu \right)}^{\lambda }+\nu^{\lambda }},\frac{2\gamma^{\lambda }}{{\left(2-\gamma \right)}^{\lambda }+\gamma^{\lambda }}\right), \end{array}$$

(8) $$\begin{array}{c} \alpha^{\lambda }=\left(\frac{2\mu^{\lambda }}{{\left(2-\mu \right)}^{\lambda }+\mu^{\lambda }},\frac{{\left(1+\nu \right)}^{\lambda }-{\left(1-\nu \right)}^{\lambda }}{{\left(1+\nu \right)}^{\lambda }+{\left(1-\nu \right)}^{\lambda }},\frac{2\gamma^{\lambda }}{{\left(2-\gamma \right)}^{\lambda }+\gamma^{\lambda }}\right). \end{array}$$

**Theorem 2 .**

Let *α*_*j*_=(*μ*_*j*_, *ν*_*j*_, *γ*_*j*_), *j* = 1, 2, and *α*=(*μ*, *ν*, *γ*) be PFVs, *λ* is a positive real number. Then, *α*_1_⊕_*ε*_*α*_2_, *α*_1_⊗_*ε*_*α*_2_, *λ*·_*ε*_*α*, and *α*^*λ*^ are also a PFV.

**Proof**

See Appendix A.

**Theorem 3 .**

Let *λ*_*j*_ ∈ [0,1], *i* *=* 1, 2, 3, and *α*=(*μ*, *ν*, *γ*) be PFVs, and *λ*_1_, *λ*_2_ and *λ* are positive real numbers, then we have the following properties:

(9) $$\begin{array}{c} \alpha_{1}{⊕}_{\varepsilon }\alpha_{2}=\alpha_{2}{⊕}_{\varepsilon }\alpha_{1}, \end{array}$$

(10) $$\begin{array}{c} \alpha_{1}{⊗}_{\varepsilon }\alpha_{2}=\alpha_{2}{⊗}_{\varepsilon }\alpha_{1}, \end{array}$$

(11) $$\begin{array}{c} \left(\alpha_{1}{⊕}_{\varepsilon }\alpha_{2}\right){⊕}_{\varepsilon }\alpha_{3}=\alpha_{1}{⊕}_{\varepsilon }\left(\alpha_{2}{⊕}_{\varepsilon }\alpha_{3}\right), \end{array}$$

(12) $$\begin{array}{c} \lambda \left(\alpha_{1}{⊕}_{\varepsilon }\alpha_{2}\right)=\lambda \alpha_{1}{⊕}_{\varepsilon }\lambda \alpha_{2}, \end{array}$$

(13) $$\begin{array}{c} {\left(\alpha_{1}{⊗}_{\varepsilon }\alpha_{2}\right)}^{\lambda }=\alpha_{1}^{\lambda }{⊗}_{\varepsilon }\alpha_{2}^{\lambda }, \end{array}$$

(14) $$\begin{array}{c} \lambda_{1}\cdot_{\varepsilon }\alpha {⊕}_{\varepsilon }\lambda_{2}\cdot_{\varepsilon }\alpha =\left(\lambda_{1}+\lambda_{2}\right)\cdot_{\varepsilon }\alpha , \end{array}$$

(15) $$\begin{array}{c} \alpha^{\lambda_{1}}{⊗}_{\varepsilon }\alpha^{\lambda_{2}}=\alpha^{\left(\lambda_{1}+\lambda_{2}\right)}. \end{array}$$

Note that the proofs of these theorems are straightforward and thus omitted here for the sake of brevity.

RETRACTED

In the next section, we investigate an Einstein hybrid aggregation operator under the picture fuzzy environment based on Einstein operations.

## 4. Picture Fuzzy Einstein Hybrid-Weighted Aggregation Operator

In this section, we propose the picture fuzzy Einstein hybrid-weighted average (PFEHWA) operator based on the proposed Einstein operations laws on picture fuzzy values.

**Definition 9 .**

Let *α*_*j*_ = (*μ*_*α*_*j*__, *ν*_*α*_*j*__, *γ*_*α*_*j*__), (*j* *=* 1, 2,…, *n*) be a collection of PFVs. The picture fuzzy Einstein hybrid-weighted average (PFIEHWA) operator is a mapping PFIEHWA : Ω^*n*^⟶Ω, with an aggregation-associated weighting vector *ω* = (*ω*_1_, *ω*_2_, ⋯,*ω*_*n*_)^*T*^, *ω*_*j*_ ∈ [0,1] and ∑_*j*=1_^*n*^*ω*_*j*_ = 1, such that

(16) $$\begin{array}{c} {\text{PFIEHWA}}_{\omega ,\lambda }\left(A_{1},A_{2},\cdots ,A_{n}\right)=\frac{\overset{n}{\underset{j=1}{{⊕}_{\varepsilon }}}\left(\omega_{\varepsilon \left(j\right)}\lambda_{j}A_{j}\right)}{\sum_{j=1}^{n}\omega_{\varepsilon \left(j\right)}\lambda_{j}}, \end{array}$$

where *ε* : (*j*)⟶(1,2, ⋯, *n*) is a permutation such that *α*_*j*_ is the *ε*(*j*)^th^ largest element of the collection of PFVs and *λ* = (*λ*_1_, *λ*_2_, ⋯,*λ*_*n*_)^*T*^ is the weighting vector of *α*_*j*_, with *λ*_*j*_ ∈ [0,1] and ∑_*j*=1_^*n*^*λ*_*j*_ = 1.

**Theorem 4 .**

For a collection of PFVs *ω*_*j*_ ∈ [0,1], *j* *=* 1, 2,…, *n*, their aggregated value by using the PFIEHWA operator is also a PFV, and

(17) $$\begin{array}{c} {\text{PFEHWA}}_{\omega ,\lambda }\left(\alpha_{1},\alpha_{2},\ldots ,\alpha_{n}\right)\\ =\left(\frac{\prod_{j=1}^{n}{\left(1+\mu_{\alpha_{j}}\right)}^{\left(\omega_{\varepsilon \left(j\right)}\lambda_{j}/\sum_{j=1}^{n}\omega_{\varepsilon \left(j\right)}\lambda_{j}\right)}-\prod_{j=1}^{n}{\left(1-\mu_{\alpha_{j}}\right)}^{\left(\omega_{\varepsilon \left(j\right)}\lambda_{j}/\sum_{j=1}^{n}\omega_{\varepsilon \left(j\right)}\lambda_{j}\right)}}{\prod_{j=1}^{n}{\left(1+\mu_{\alpha_{j}}\right)}^{\left(\omega_{\varepsilon \left(j\right)}\lambda_{j}/\sum_{j=1}^{n}\omega_{\varepsilon \left(j\right)}\lambda_{j}\right)}+\prod_{j=1}^{n}{\left(1-\mu_{\alpha_{j}}\right)}^{\left(\omega_{\varepsilon \left(j\right)}\lambda_{j}/\sum_{j=1}^{n}\omega_{\varepsilon \left(j\right)}\lambda_{j}\right)}},\right.\\ \frac{2\prod_{j=1}^{n}{\left(\nu_{\alpha_{j}}\right)}^{\left(\omega_{\varepsilon \left(j\right)}\lambda_{j}/\sum_{j=1}^{n}\omega_{\varepsilon \left(j\right)}\lambda_{j}\right)}}{\prod_{j=1}^{n}{\left(2-\left(\nu_{\alpha_{j}}\right)\right)}^{\left(\omega_{\varepsilon \left(j\right)}\lambda_{j}/\sum_{j=1}^{n}\omega_{\varepsilon \left(j\right)}\lambda_{j}\right)}+\prod_{j=1}^{n}{\left(\nu_{\alpha_{j}}\right)}^{\left(\omega_{\varepsilon \left(j\right)}\lambda_{j}/\sum_{j=1}^{n}\omega_{\varepsilon \left(j\right)}\lambda_{j}\right)}},\\ \left.\frac{2\prod_{j=1}^{n}{\left(\gamma_{\alpha_{j}}\right)}^{\left(\omega_{\varepsilon \left(j\right)}\lambda_{j}/\sum_{j=1}^{n}\omega_{\varepsilon \left(j\right)}\lambda_{j}\right)}}{\prod_{j=1}^{n}{\left(2-\left(\gamma_{\alpha_{j}}\right)\right)}^{\left(\omega_{\varepsilon \left(j\right)}\lambda_{j}/\sum_{j=1}^{n}\omega_{\varepsilon \left(j\right)}\lambda_{j}\right)}+\prod_{j=1}^{n}{\left(\gamma_{\alpha_{j}}\right)}^{\left(\omega_{\varepsilon \left(j\right)}\lambda_{j}/\sum_{j=1}^{n}\omega_{\varepsilon \left(j\right)}\lambda_{j}\right)}}\right). \end{array}$$

**Proof**

See Appendix B.

RETRACTED

**Theorem 5 .**

The PFIEHWA operator satisfies the following properties:

(1) (Idempotency): If *α*_*j*_=(*μ*_*α*_*j*__, *ν*_*α*_*j*__, *γ*_*α*_*j*__),  *j*=1,2,…, *n* are all equal, that is, *α*_*j*_=*α*, for all *j*=1,2,…, *n*. Then,
  (18) $$\begin{array}{c} {\text{PFIEHWA}}_{\omega ,\lambda }\left(\alpha_{1},\alpha_{2},\ldots ,\alpha_{n}\right)=\alpha . \end{array}$$
(2) (Boundedness): Let $\alpha_{\min}=\left(\underset{1\leq j\leq n}{\min}\mu_{\alpha_{j}},\underset{1\leq j\leq n}{\max}\nu_{\alpha_{j}},\underset{1\leq j\leq n}{\max}\gamma_{\alpha_{j}}\right)$ and $\alpha_{\max}=\left(\underset{1\leq j\leq n}{\max}\mu_{\alpha_{j}},\underset{1\leq j\leq n}{\min}\nu_{\alpha_{j}},\underset{1\leq j\leq n}{\min}\gamma_{\alpha_{j}}\right)$, then
  (19) $$\begin{array}{c} \alpha_{\min}\leq {\text{PFIEHWA}}_{\omega ,\lambda }\left(\alpha_{1},\alpha_{2},\ldots ,\alpha_{n}\right)\leq \alpha_{\max}. \end{array}$$
(3) (Monotonicity): Let *α*_*j*_^1^=(*μ*_*α*_*j*__^1^, *ν*_*α*_*j*__^1^, *γ*_*α*_*j*__^1^),  *j*=1,2,…, *n* and *α*_*j*_^2^=(*μ*_*α*_*j*__^2^, *ν*_*α*_*j*__^2^, *γ*_*α*_*j*__^2^), *j* = 1, 2,…, *n*, be two collections of PFVs, if *μ*_*α*_*j*__^1^ ≤ *μ*_*α*_*j*__^2^, *ν*_*α*_*j*__^1^ ≥ *ν*_*α*_*j*__^2^, and *γ*_*α*_*j*__^1^ ≥ *γ*_*α*_*j*__^2^. Then,
  (20) $$\begin{array}{c} {\text{PFIEHWA}}_{\omega ,\lambda }\left(\alpha_{1}^{1},\alpha_{2}^{1},\ldots ,\alpha_{n}^{1}\right)\leq {\text{PFEIHWA}}_{\omega ,\lambda }\left(\alpha_{1}^{2},\alpha_{2}^{2},\ldots ,\alpha_{n}^{2}\right). \end{array}$$

**Proof**

See Appendix C.

RETRACTED

## 5. Application of Picture Einstein Fuzzy Hybrid Aggregation Operator

In this section, we investigate the application of the picture Einstein fuzzy hybrid aggregation operator in group decision making with picture fuzzy information.

### 5.1. MAGDM Method Based on the PFIEHWA Operator

For a MCGMD problem under the picture fuzzy environment, let *D*=(*d*_1_,*d*_2_, ⋯ ,*d*_*l*_) be a set of decision makers, *C*=(*C*_1_, *C*_2_, ⋯, *C*_*n*_) be a set of criteria, and *X*=(*X*_1_, *X*_2_, ⋯, *X*_*m*_) be a set of alternatives to be evaluated. Let ${\tilde{D}}^{\left(k\right)}={\left({\tilde{\alpha }}_{ij}^{\left(k\right)}\right)}_{m\times n}$ be a picture fuzzy decision matrix, where ${\tilde{\alpha }}_{ij}^{\left(k\right)}=\left(\mu_{\alpha_{ij}}^{\left(k\right)},\nu_{\alpha_{ij}}^{\left(k\right)},\gamma_{\alpha_{ij}}^{\left(k\right)}\right)$ is a PFV for alternative *X*_*i*_ with respect to criteria *C*_*j*_ provided by decision maker *d*_*k*_, such that 0 ≤ *μ*_*α*_*ij*__^(*k*)^ ≤ 1, 0 ≤ *ν*_*α*_*ij*__^(*k*)^ ≤ 1, 0 ≤ *γ*_*α*_*ij*__^(*k*)^ ≤ 1, 0 ≤ *μ*_*α*_*ij*__^(*k*)^+*ν*_*α*_*ij*__^(*k*)^+*γ*_*α*_*ij*__^(*k*)^ ≤ 1, *k*=1,2, ⋯, *l*, *i*=1,2, ⋯, *m* and *j*=1,2, ⋯, *n*. The expert committee gives the weighting vector *λ*=(*λ*^(1)^, *λ*^(2)^, ⋯,*λ*^(*l*)^)^*T*^ for the decision makers, where *λ*^(*k*)^ ∈ [0,1] and ∑_*k*=1_^*l*^*λ*^(*k*)^=1. Considering that different decision makers are familiar with differentiated fields, the expert committee also determines the ordering weights vector *ω*=(*ω*^(1)^, *ω*^(2)^, ⋯,*ω*^(*l*)^)^*T*^ for the decision makers, where *ω*^(*k*)^ ∈ [0,1]and ∑_*k*=1_^*l*^*ω*^(*k*)^=1. After that, the picture fuzzy decision matrixes ${\tilde{D}}^{\left(k\right)}={\left({\tilde{\alpha }}_{ij}^{\left(k\right)}\right)}_{m\times n}$ will be aggregated into a collective picture fuzzy decision matrix $\tilde{D}={\left({\tilde{\alpha }}_{ij}\right)}_{m\times n}$. Then, the expert committee assigns the weighting vector *η*=(*η*_1_, *η*_2_, ⋯,*η*_*n*_)^*T*^ for the criteria according to their relative importance in decision making, where *η*_*j*_ ∈ [0,1] and ∑_*j*=1_^*n*^*η*_*j*_=1. Meanwhile, considering the fact that diverse alternatives may have differentiated focuses and advantages, the expert committee also gives the aggregation-associated weights vector *ξ*=(*ξ*_1_, *ξ*_2_, ⋯,*ξ*_*n*_)^*T*^ for different criteria, where *ξ*_*j*_ ∈ [0,1] and ∑_*j*=1_^*n*^*ξ*_*j*_=1.

RETRACTED

The complete procedure for multicriteria group decision making based on the proposed picture fuzzy Einstein hybrid-weighted aggregation operator can be summarized as follows:

**Step 1 .**

In order to eliminate the impact of different types of criteria values (i.e., benefit criteria or cost criteria), we will transform the criteria values of cost type into those of the benefit type i.e., transform ${\tilde{D}}^{\left(k\right)}={\left({\tilde{\alpha }}_{ij}^{\left(k\right)}\right)}_{m\times n}$ into a normalized picture fuzzy decision matrix ${\tilde{R}}^{\left(k\right)}={\left({\tilde{r}}_{ij}^{\left(k\right)}\right)}_{m\times n}$, where

(21) $$\begin{array}{c} {\tilde{r}}_{ij}^{\left(k\right)}=\left\{\begin{array}{cc} \alpha_{ij}^{k} & \mathrm{for}\;\mathrm{benefit}\;\mathrm{criteria}\\ {\left(\alpha_{ij}^{k}\right)}^{c} & \mathrm{for}\;\mathrm{cost}\;\mathrm{criteria} \end{array}\right., \end{array}$$

where (*α*_*ij*_^*k*^)^*c*^ is the complement of *α*_*ij*_^*k*^ such that (*α*_*ij*_^*k*^)^*c*^ = (*ν*_*ij*_^(*k*)^, *μ*_*ij*_^(*k*)^, *γ*_*ij*_^(*k*)^).

**Step 2 .**

Utilizing the *PFIEHWA* operator to aggregate picture fuzzy decision matrixes ${\tilde{R}}^{\left(k\right)}={\left({\tilde{r}}_{ij}^{\left(k\right)}\right)}_{m\times n}$ into a collective picture fuzzy decision matrix $\tilde{R}={\left({\tilde{r}}_{i}^{\left(k\right)}\right)}_{m\times k}$.

(22) $$\begin{array}{c} {\tilde{r}}_{i}^{\left(k\right)}={\text{PFIEHWA}}_{\omega ,\lambda }\left({\tilde{r}}_{i1}^{\left(k\right)},{\tilde{r}}_{i2}^{\left(k\right)},\cdots ,{\tilde{r}}_{in}^{\left(k\right)}\right)=\overset{n}{\underset{j=1}{{⊕}_{\varepsilon }}}\frac{\left(\xi_{\varepsilon \left(ij\right)}^{\left(k\right)}\lambda_{j}{\tilde{r}}_{ij}^{\left(k\right)}\right)}{\sum_{k=1}^{l}\xi_{\varepsilon \left(ij\right)}^{\left(k\right)}\lambda_{j}}. \end{array}$$

**Step 3 .**

Utilizing the *PFIEHWA*${\tilde{r}}_{i}$ to aggregate all the evaluation values ${\tilde{r}}_{i}^{\left(k\right)}$ into a collective evaluation value ${\tilde{r}}_{i}$ for alternative*X*_*i*_.

(23) $$\begin{array}{c} {\tilde{r}}_{i}={\text{PFIEHWA}}_{\xi ,\eta }\left({\tilde{r}}_{i}^{\left(1\right)},{\tilde{r}}_{i}^{\left(2\right)},{\tilde{r}}_{i}^{\left(3\right)},\cdots ,{\tilde{r}}_{i}^{\left(l\right)}\right)=\overset{l}{\underset{k=1}{{⊕}_{\varepsilon }}}\frac{\left(\omega_{\varepsilon \left(ik\right)}\eta_{k}{\tilde{r}}_{i}^{\left(k\right)}\right)}{\sum_{k=1}^{l}\omega_{\varepsilon \left(ik\right)}\eta_{k}}. \end{array}$$

**Step 4 .**

RETRACTED

Ranking${\tilde{r}}_{i}$ by using the ranking method described in Section 2 and select the best one.

### 5.2. Illustrative Example

In this section, we use an example presented in [49] to illustrate the proposed method.

**Example 1 (49).**

Suppose a company wants to develop a new career, where there are three alternatives: *X*_1_, *X*_2_, and *X*_3_ to be selected. *X*_1_ is the real estate industry, *X*_2_ is the food industry, and *X*_3_ is the education industry. After preliminary screening, three experts *d*_1_, *d*_2_, and *d*_3_ are asked to evaluate the alternatives. Four criteria are determined: the ability to compete (*C*_1_), the ability to grow (*C*_2_), the influence of the surrounding environment (*C*_3_), and the influence of social politics (*C*_4_). Assume that the subjective importance degree of each decision maker is *λ* = (0.2, 0.4, 0.4)^*T*^. Simultaneously, considering that some decision makers could be more familiar with career management, the aggregation-associated weighting vector of decision maker *d*_*k*_ is *ω* = (0.3, 0.3, 0.4)^*T*^. Furthermore, suppose the weight vector and aggregation -associated weight vector for the four criteria are *η* = (0.2, 0.3, 0.3, 0.2)^*T*^ and *ξ* = (0.2, 0.1, 0.3, 0.4)^*T*^, respectively. The picture fuzzy decision matrices are given as follows:

(24) $$\begin{array}{c} {\tilde{D}}^{\left(1\right)}=\left[\begin{array}{cccc} \left(0.1,0.3,0.5\right) & \left(0.5,0.2,0.3\right) & \left(0.2,0.2,0.1\right) & \left(0.3,0.1,0.2\right)\\ \left(0.2,0.2,0.3\right) & \left(0.1,0.2,0.4\right) & \left(0.2,0.1,0.3\right) & \left(0.1,0.2,0.3\right)\\ \left(0.1,0.3,0.5\right) & \left(0.3,0.1,0.2\right) & \left(0.3,0.2,0.1\right) & \left(0.2,0.3,0.2\right) \end{array}\right],\\ {\tilde{D}}^{\left(2\right)}=\left[\begin{array}{cccc} \left(0.3,0.1,0.2\right) & \left(0.3,0.1,0.2\right) & \left(0.3,0.1,0.2\right) & \left(0.2,0.2,0.3\right)\\ \left(0.1,0.3,0.2\right) & \left(0.2,0.1,0.3\right) & \left(0.3,0.3,0.2\right) & \left(0.3,0.1,0.1\right)\\ \left(0.2,0.3,0.1\right) & \left(0.2,0.1,0.3\right) & \left(0.4,0.1,0.3\right) & \left(0.2,0.1,0.3\right) \end{array}\right],\\ {\tilde{D}}^{\left(3\right)}=\left[\begin{array}{cccc} \left(0.5,0.1,0.1\right) & \left(0.5,0.2,0.1\right) & \left(0.2,0.4,0.1\right) & \left(0.3,0.1,0.1\right)\\ \left(0.4,0.1,0.2\right) & \left(0.3,0.2,0.4\right) & \left(0.2,0.1,0.4\right) & \left(0.5,0.2,0.1\right)\\ \left(0.4,0.2,0.2\right) & \left(0.4,0.2,0.1\right) & \left(0.5,0.2,0.3\right) & \left(0.3,0.2,0.3\right) \end{array}\right]. \end{array}$$

**Step 5 .**

Considering the criteria are all the benefit criteria, there is no need to transform them into benefits ones. Thus we have${\tilde{D}}^{\left(k\right)}={\tilde{R}}^{\left(k\right)}$

**Step 6 .**

RETRACTED

Utilizing the PFIEHWA operator to aggregate all individual picture fuzzy decision matrixes ${\tilde{R}}^{\left(k\right)}$into a collective picture fuzzy decision matrix $\tilde{R}$

(1 − *μ*_*A*_*j*__^1^)/(1 − *μ*_*A*_*j*__^1^) ≤ (1+*μ*_*A*_*j*__^2^)/(1+*μ*_*A*_*j*__^2^)

Let us illustrate this step by using ${\tilde{r}}_{11}$ as an example. Since ${\tilde{r}}_{\mathrm{11}}^{\left(1\right)}=\left(0.1,0.3,0.5\right)$, ${\tilde{r}}_{12}^{\left(1\right)}=\left(0.5,0.2,0.3\right)$, ${\tilde{r}}_{13}^{\left(1\right)}=\left(0.2,0.2,0.1\right)$， ${\tilde{r}}_{14}^{\left(4\right)}=\left(0.3,0.2,0.1\right)$, *η* = (0.2, 0.3, 0.3, 0.2)^*T*^, and *ξ* = (0.2, 0.1, 0.3, 0.4)^*T*^, we have $S\left({\tilde{r}}_{11}^{\left(1\right)}\right)=-0.2$, $S\left({\tilde{r}}_{12}^{\left(1\right)}\right)=0.3$, $S\left({\tilde{r}}_{13}^{\left(1\right)}\right)=0$, and $S\left({\tilde{r}}_{14}^{\left(1\right)}\right)=0.1$ by using the ranking function given in Theorem 1. Thus, we can obtain $S\left({\tilde{r}}_{11}^{\left(1\right)}\right)<S\left({\tilde{r}}_{13}^{\left(1\right)}\right)<S\left({\tilde{r}}_{14}^{\left(1\right)}\right)<S\left({\tilde{r}}_{12}^{\left(1\right)}\right)$, which implies that ${\tilde{r}}_{11}^{\left(1\right)}<\left.{\tilde{r}}_{13}^{\left(1\right)}\right)<{\tilde{r}}_{14}^{\left(1\right)}<{\tilde{r}}_{12}^{\left(1\right)}$. Hence, we have *ε*_11_(1) = 4, *ε*_12_(1) = 3, *ε*_13_(1) = 2, and *ε*_14_(1) = 1. Then,

(25) $$\begin{array}{c} \frac{\xi_{\varepsilon_{11}\left(1\right)}\eta_{1}^{\left(1\right)}}{\sum_{j=1}^{4}\xi_{\varepsilon_{1j}}^{{}_{\left(1\right)}}\eta_{1}^{\left(1\right)}}=\frac{0.2\times 0.4}{0.2\times 0.4+0.3\times 0.3+0.3\times 0.1+0.2\times 0.2}=0.3333\text{,}\\ \frac{\xi_{\varepsilon_{12}\left(1\right)}\eta_{2}^{\left(1\right)}}{\sum_{j=1}^{4}\xi_{\varepsilon_{1j}\left(1\right)}\eta_{2}^{\left(1\right)}}=\frac{0.3\times 0.3}{0.2\times 0.4+0.3\times 0.3+0.3\times 0.1+0.2\times 0.2}=0.3750,\\ \frac{\xi_{\varepsilon_{13}\left(1\right)}\eta_{3}^{\left(1\right)}}{\sum_{j=1}^{4}\xi_{\varepsilon_{1j}}^{\left(1\right)}\eta_{3}^{\left(1\right)}}=\frac{0.3\times 0.1}{0.2\times 0.4+0.3\times 0.3+0.3\times 0.1+0.2\times 0.2}=0.1250,\\ \frac{\xi_{\varepsilon_{14}\left(1\right)}\eta_{4}^{\left(1\right)}}{\sum_{j=1}^{4}\xi_{\varepsilon_{1j}}^{\left(1\right)}\eta_{4}^{\left(1\right)}}=\frac{0.2\times 0.2}{0.2\times 0.4+0.3\times 0.3+0.3\times 0.1+0.2\times 0.2}=0.1667\text{.} \end{array}$$

Finally, we have $PFIEHWA_{\xi ,\eta }\left({\tilde{r}}_{11}^{\left(1\right)},{\tilde{r}}_{12}^{\left(1\right)},{\tilde{r}}_{13}^{\left(1\right)},{\tilde{r}}_{14}^{\left(1\right)}\right)=\left(0.1720,0.2054,0.2958\right)$ by using (21). Similarly, we can derive the collective evaluation matrix given in Table 1.

RETRACTED

**Step 7 .**

Utilizingthe *PFIEHWA* operator to aggregate all ${\tilde{r}}_{i}^{\left(k\right)}$, *k* *=* 1, 2, 3, into a collective PFV ${\tilde{r}}_{i}$ for alternative *X*_*i*_ over all the experts. According to Theorem 1, we have $S\left({\tilde{r}}_{1}^{\left(1\right)}\right)=-0.0334$, $S\left({\tilde{r}}_{1}^{\left(2\right)}\right)=-0.1$ and $S\left({\tilde{r}}_{1}^{\left(3\right)}\right)=-0.0376$. Thus, $S\left({\tilde{r}}_{1}^{\left(3\right)}\right)<S\left({\tilde{r}}_{1}^{\left(1\right)}\right)<S\left({\tilde{r}}_{1}^{\left(2\right)}\right)$, which means that ${\tilde{r}}_{1}^{\left(3\right)}<{\tilde{r}}_{1}^{\left(1\right)}<{\tilde{r}}_{1}^{\left(2\right)}$. Hence, *δ*_11_ = 2, *δ*_12_ = 3 and *δ*_13_ = 1. Then, we have as follows:

(26) $$\begin{array}{c} \omega_{\varepsilon \left(11\right)}\frac{\lambda_{1}}{\sum_{k=1}^{3}\omega_{\varepsilon_{\left(1k\right)}}\lambda_{k}}=\frac{\left(0.2\times 0.3\right)}{\left(0.2\times 0.3+0.4\times 0.3+0.4\times 0.4\right)}=0.1765\text{,}\\ \omega_{\varepsilon \left(12\right)}\frac{\lambda_{2}}{\sum_{k=1}^{3}\omega_{\varepsilon_{\left(1k\right)}}\lambda_{k}}=\frac{\left(0.4\times 0.3\right)}{\left(0.2\times 0.3+0.4\times 0.3+0.4\times 0.4\right)}=0.3529\text{,}\\ \omega_{\varepsilon \left(13\right)}\frac{\lambda_{3}}{\sum_{k=1}^{3}\omega_{\varepsilon_{\left(1k\right)}}\lambda_{k}}=\frac{\left(0.4\times 0.4\right)}{\left(0.2\times 0.3+0.4\times 0.3+0.4\times 0.4\right)}=0.4706\text{.} \end{array}$$

Thus, we can derive the following result:

(27) $$\begin{array}{c} {\tilde{r}}_{1}={\text{PFIEHWA}}_{\omega ,\lambda }\left({\tilde{r}}_{1}^{\left(1\right)},{\tilde{r}}_{2}^{\left(1\right)},{\tilde{r}}_{3}^{\left(1\right)},{\tilde{r}}_{4}^{\left(1\right)}\right)=\left(0.1129\text{, }0.1650\text{, }0.2894\right). \end{array}$$

Similarly, we can obtain the following results:

(28) $$\begin{array}{c} {\tilde{r}}_{2}={\text{PFIEHWA}}_{\omega ,\lambda }\left({\tilde{r}}_{1}^{\left(2\right)},{\tilde{r}}_{2}^{\left(2\right)},{\tilde{r}}_{3}^{\left(2\right)},{\tilde{r}}_{4}^{\left(2\right)}\right)=\left(0.1156\text{,}0.1424\text{,}0.2271\right)\text{,}\\ {\tilde{r}}_{3}={\text{PFIEHWA}}_{\omega ,\lambda }\left({\tilde{r}}_{1}^{\left(3\right)},{\tilde{r}}_{2}^{\left(3\right)},{\tilde{r}}_{3}^{\left(3\right)},{\tilde{r}}_{4}^{\left(3\right)}\right)=\left(0.1812\text{,}0.1639\text{,}0.1821\right). \end{array}$$

**Step 8 .**

Computingthe ranking values $R\left({\tilde{r}}_{i}\right)$ for *A*_*i*_, for all *k* *=* 1, 2, and 3. By using Theorem 1, we have $S\left({\tilde{r}}_{1}\right)=-0.0521$, $S\left({\tilde{r}}_{2}\right)=-0.0268$, and $S\left({\tilde{r}}_{3}\right)=0.0173$. Since $S\left({\tilde{r}}_{1}\right)<S\left({\tilde{r}}_{2}\right)<S\left({\tilde{r}}_{3}\right)$, we obtain *X*_1_ < *X*_2_ < *X*_3_, which implies that *X*_3_ is the most desirable career alternative. This order is the same as the method proposed by Liu and Shi's work.

RETRACTED

### 5.3. Comparative Analysis

In this section, we compare the proposed method based on the *PFEHWA* operator with the method given by Zhang [44], Peng [56], and Liu [48] using the following example in [44]. In the method proposed by Zhang [44], a quasi-intuitionistic fuzzy Einstein hybrid-weighted averaging (*QIFEHWA*) operator and intuitionistic fuzzy Einstein weighted averaging (*IFEWA*) operator were utilized, which does not consider hesitation or neutral information in the aggregation process, whereas the method given by Peng [56], Liu [48], and the proposed method considers hesitation or neutral information. In the method of Peng [56] and Liu [48], NS was used to develop some single-valued Neutrosophic fuzzy-weighted averaging operators, such as the Einstein single-valued neutrosophic number-weighted averaging (*ESVNNWA*) operator in [48] and the simplified neutrosophic hybrid ordered weighted averaging (*SNNHOWA*) operator in [56].

**Example 2 (44).**

Suppose a computer center in a university wants to select a new information system from the following four possible alternatives: *X*_1_*, X*_2_*, X*_3_, and *X*_4_. Three decision makers are asked to make a decision according to the following four criteria: (1) *C*_1_ is the costs of the hardware and software investment; (2) *C*_2_ is the contribution to organization performance; (3) *C*_3_ is the effort to transition from the current systems; and (4) *C*_4_ is the reliability of outsourcing software development; these are all benefit type criteria. Suppose the weights vector of decision makers *d*_1_, *d*_2_, and *d*_3_ is *λ*=(*λ*^1^, *λ*^2^, *λ*^3^)^*T*^=(0.2, 0.5, 0.3)^*T*^ and the associated-weighting vector is *ω*=(*ω*^1^, *ω*^2^, *ω*^3^)^*T*^=(1/3, 1/3, 1/3)^*T*^. Then, the decision maker *d*_*k*_ determines the weight vector of four criteria, which are *η*_*j*_^(1)^=(0.4, 0.3, 0.1, 0.2)^*T*^, *η*_*j*_^(2)^=(0.1, 0.3, 0.5, 0.1)^*T*^, and *η*_*j*_^(3)^=(0.1, 0.2, 0.3, 0.4)^*T*^, where *j*=1,2,3,4. According to their preferences, the decision makers also give the associated-weighting vectors of the four criteria: *ξ*_*j*_^(1)^=(0.4, 0.3, 0.2, 0.1)^*T*^, *ξ*_*j*_^(2)^=(0.3, 0.3, 0.2, 0.2)^*T*^, and *ξ*_*j*_^(3)^=(0.5, 0.3, 0.1, 0.1)^*T*^, where *j*=1,2,3,4. Considering that the value of each criterion is evaluated using the intuitionistic fuzzy information by the decision makers, we first transform IFVs into PFVs, as shown in Tables 2-4.

RETRACTED

A comparison of the ranking results using different methods is shown in Table 5. We can see from Table 5 that different methods lead to different rankings. However, *X*_2_ is always the best alternative. We can also see that the method of Liu and our method generate the same ranking for four alternatives. The reason can be explained as follows. First, the shortcomings of IFSs and NSs that were discussed earlier can account for the differences in the final rankings. Second, these methods apply different types of ranking measures to rank IFSs or NSs, such as the score function or accuracy function. In the proposed method, a novel ranking function based on the parametric distance measure can distinguish two different PFVs while other ranking measures could not.

## 6. Conclusion

In this study, we have proposed a hybrid Einstein aggregation operator on the basis of the proposed picture Einstein operations for aggregating picture fuzzy information and investigated their application in multicriteria group decision making. First, based on the picture Einstein operation laws, we have developed a new operator for aggregating PFVs. Then, we have utilized the proposed operator to develop a method for MCGDM problems in which the evaluation values are represented by PFVs. Finally, an example is conducted to illustrate the practicality and effectiveness of the proposed MCGDM approach. In future research, the proposed method could be extended to interval-valued picture fuzzy sets and trapezoidal picture fuzzy sets. Another interesting direction could be to develop other types of picture fuzzy aggregation operators.

## Figures and Tables

**Table 1:** Collective picture fuzzy decision matrix.

	*D*_1_	*D*_2_	*D*_3_
*X*_1_	(0.1720, 0.2054, 0.2958)	(0.1355, 0.1265, 0.2296)	(0.1728, 0.1879, 0.100)
*X*_2_	(0.0700, 0.1700, 0.3334)	(0.1057, 0.1679, 0.2090)	(0.1655, 0.1219, 0.2764)
*X*_3_	(0.1109, 0.1485, 0.2575)	(0.1174, 0.1210, 0.2522)	(0.2007, 0.2000, 0.1753)

**Table 2:** Picture fuzzy decision matrix ${\tilde{D}}^{\left(1\right)}$.

	*C*_1_	*C*_2_	*C*_3_	*C*_4_
*X*_1_	(0.5, 0.4, 0.1)	(0.4, 0.3, 0.3)	(0.5, 0.3, 0.2)	(0.2, 0.6, 0.2)
*X*_2_	(0.5, 0.4, 0.1)	(0.3, 0.7, 0.0)	(0.2, 0.8, 0.0)	(0.4, 0.5, 0.1)
*X*_3_	(0.2, 0.6, 0.2)	(0.8, 0.1, 0.1)	(0.6, 0.4, 0.0)	(0.1, 0.7, 0.2)
*X*_4_	(0.1, 0.9, 0.0)	(0.2, 0.8, 0.0)	(0.7, 0.2, 0.1)	(0.4, 0.6, 0.0)

**Table 3:** Picture fuzzy decision matrix ${\tilde{D}}^{\left(2\right)}$.

	*C*_1_	*C*_2_	*C*_3_	*C*_4_
*X*_1_	(0.3, 0.6, 0.1)	(0.2, 0.7, 0.1)	(0.5, 0.5, 0.0)	(0.5, 0.3, 0.2)
*X*_2_	(0.3, 0.7, 0.0)	(0.6, 0.4, 0.0)	(0.7, 0.2, 0.1)	(0.4, 0.5, 0.1)
*X*_3_	(0.6, 0.3, 0.1)	(0.4, 0.4, 0.2)	(0.2, 0.7, 0.1)	(0.3, 0.6, 0.1)
*X*_4_	(0.2, 0.5, 0.3)	(0.5, 0.3, 0.2)	(0.5, 0.4, 0.1)	(0.4, 0.3, 0.3)

RETRACTED

**Table 4:** Picture fuzzy decision matrix ${\tilde{D}}^{\left(3\right)}$.

	*C*_1_	*C*_2_	*C*_3_	*C*_4_
*X*_1_	(0.7, 0.3, 0.0)	(0.4, 0.5, 0.1)	(0.5, 0.4, 0.1)	(0.6, 0.2, 0.2)
*X*_2_	(0.5, 0.5, 0.0)	(0.3, 0.5, 0.2)	(0.8, 0.1, 0.1)	(0.7, 0.1, 0.2)
*X*_3_	(0.8, 0.2, 0.0)	(0.2, 0.3, 0.5)	(0.6, 0.3, 0.1)	(0.2, 0.7, 0.1)
*X*_4_	(0.9, 0.1, 0.0)	(0.8, 0.1, 0.1)	(0.2, 0.1, 0.7)	(0.2, 0.6, 0.2)

**Table 5:** Ranking results for example 2.

Methods	Ranking values	Ranking results
Zhang method [44] (QIFEHWA and IFEWA operator)	S(*r*_*1*_) = 0.0913; S(*r*_*2*_) = 0.3768; S(*r*_*3*_) = 0.0736; S(*r*_*4*_) = 0.1769.	*X*_2_≻*X*_4_≻*X*_1_≻*X*_3_
Peng method [58] (SNNHOWA operator)	S(*r*_*1*_) = 0.7609; S(*r*_*2*_) = 0.8456; S(*r*_*3*_) = 0.7281; S(*r*_*4*_) = 0.7577.	*X*_2_≻*X*_1_≻*X*_4_≻*X*_3_
Liu method [48] (ESVNNWA operator)	S(*r*_*1*_) = 0.6486; S(*r*_*2*_) = 0.7550; S(*r*_*3*_) = 0.6519; S(*r*_*2*_) = 0.6912.	*X*_2_≻*X*_4_≻*X*_3_≻*X*_1_
Our method (PFEHWA operator)	S(*r*_*1*_) = 0.4655; S(*r*_*2*_) = 0.6142; S(*r*_*3*_) = 0.5080; S(*r*_*2*_) = 05543.	*X*_2_≻*X*_4_≻*X*_3_≻*X*_1_

## Data Availability

The data used to support the findings of this study are included within the article.

## Appendix

### A. Proof of Theorem 2

Proof We first proof that *α*_1_⊕_*ε*_*α*_2_ is a PFV. Since 0 ≤ *μ*_1_, *μ*_2_, *ν*_1_, *ν*_2_, *γ*_1_, *γ*_2_ ≤ 1, 0 ≤ *μ*_1_+*ν*_1_+*γ*_1_ ≤ 1 and 0 ≤ *μ*_2_+*ν*_2_+*γ*_2_ ≤ 1, we obtain 1 − *ν*_1_ ≥ *μ*_1_, 1 − *ν*_2_ ≥ *μ*_2_, 1 − *γ*_1_ ≥ *μ*_1_, and 1 − *γ*_2_ ≥ *μ*_2_. Thus, we have as follows:

(A.1) $$\begin{array}{c} \frac{\mu_{1}+\mu_{2}}{1+\mu_{1}\mu_{2}}+\frac{\nu_{1}\nu_{2}}{1+\left(1-\nu_{1}\right)\left(1-\nu_{2}\right)}+\frac{\gamma_{1}\gamma_{2}}{1+\left(1-\gamma_{1}\right)\left(1-\gamma_{2}\right)}\leq \frac{\mu_{1}+\mu_{2}}{1+\mu_{1}\mu_{2}}+\frac{\nu_{1}\nu_{2}}{1+\mu_{1}\mu_{2}}+\frac{\gamma_{1}\gamma_{2}}{1+\mu_{1}\mu_{2}}\\ =\frac{\mu_{1}+\mu_{2}+\nu_{1}\nu_{2}+\gamma_{1}\gamma_{2}}{1+\mu_{1}\mu_{2}}\\ \leq \frac{\mu_{1}+\mu_{2}+\left(1-\left(\mu_{1}+\gamma_{1}\right)\right)\left(1-\left(\mu_{2}+\gamma_{2}\right)\right)+\gamma_{1}\gamma_{2}}{1+\mu_{1}\mu_{2}}\\ \leq \frac{1-\left(\mu_{1}+\mu_{2}+\mu_{1}\mu_{2}+\mu_{1}\gamma_{2}+\mu_{2}\gamma_{1}\right)}{1+\mu_{1}\mu_{2}}\leq 1, \end{array}$$

that is, to say, *α*_1_⊕_*ε*_*α*_2_ is a PFV. Similarly, we can prove that *α*_1_⊗_*ε*_*α*_2_ is also a PFV. We now prove that *λ*·_*ε*_*α* is a PFV. To achieve this purpose, we first prove that *m*·_*ε*_*α* is a PFV for any arbitrary positive integer. Let *m* be any positive integer and *α* is a PFV, then

(A.2) $$\begin{array}{c} m\cdot_{\varepsilon }\alpha =\overset{m}{\overset{︷}{\alpha {⊕}_{\varepsilon }\alpha {⊕}_{\varepsilon }\cdots {⊕}_{\varepsilon }\alpha }}. \end{array}$$

Now, we prove that equation (7) holds for all positive integers with induction method. First of all, we prove that equation (7) holds for *m* = 1. Since

(A.3) $$\begin{array}{c} 1\cdot_{\varepsilon }\alpha =\left(\frac{{\left(1+\mu \right)}^{1}-{\left(1-\mu \right)}^{1}}{{\left(1+\mu \right)}^{1}+{\left(1-\mu \right)}^{1}},\frac{2\nu^{1}}{{\left(2-\nu \right)}^{1}+\nu^{1}},\frac{2\gamma^{1}}{{\left(2-\gamma \right)}^{1}+\gamma^{1}}\right)\\ =\left(\mu ,\nu ,\gamma \right)=\alpha . \end{array}$$

Therefore, equation (7) holds for *m=*1. Second, if equation (7) holds for *m=k*, that is to say

(A.4) $$\begin{array}{c} k\cdot_{\varepsilon }\alpha =\overset{k}{\overset{︷}{\alpha {⊕}_{\varepsilon }\alpha {⊕}_{\varepsilon }\cdots {⊕}_{\varepsilon }\alpha }}. \end{array}$$

When *m=k+*1, we have the following:

(A.5) $$\begin{array}{c} \overset{k+1}{\overset{︷}{\alpha {⊕}_{\varepsilon }\alpha {⊕}_{\varepsilon }\cdots {⊕}_{\varepsilon }\alpha }}=\overset{k}{\overset{︷}{\alpha {⊕}_{\varepsilon }\alpha {⊕}_{\varepsilon }\cdots {⊕}_{\varepsilon }\alpha }}{⊕}_{\varepsilon }\alpha ,\\ =\left(\frac{{\left(1+\mu \right)}^{k}-{\left(1-\mu \right)}^{k}}{{\left(1+\mu \right)}^{k}+\left({\left(1-\mu \right)}^{k}\right.},\frac{2\nu^{k}}{{\left(2-\nu \right)}^{k}+\nu^{k}},\frac{2\gamma^{k}}{{\left(2-\gamma \right)}^{k}+\gamma^{k}}\right){⊕}_{\varepsilon }\left(\mu ,\nu ,\gamma \right),\\ =\left(\frac{{\left(1+\mu \right)}^{k}-{\left(1-\mu \right)}^{k}}{{\left(1+\mu \right)}^{k}+{\left(1-\mu \right)}^{k}},\frac{2\nu^{k}}{{\left(2-\nu \right)}^{k}+\nu^{k}},\frac{2\gamma^{k}}{{\left(2-\gamma \right)}^{k}+\gamma^{k}}\right){⊕}_{\varepsilon }\left(\frac{\left(1+\mu \right)-\left(1-\mu \right)}{\left(1+\mu \right)+\left(1-\mu \right)},\frac{2\nu }{\left(2-\nu \right)+\nu },\frac{2\gamma }{\left(2-\gamma \right)+\gamma }\right),\\ \left.\frac{2\gamma^{k}/{\left(2-\gamma \right)}^{k}+\gamma^{k}\times 2\gamma /\left(2-\gamma \right)+\gamma }{1+\left(1-2\gamma^{k}/{\left(2-\gamma \right)}^{k}+\gamma^{k}\right)\left(1-2\gamma /\left(2-\gamma \right)+\gamma \right)}\right),\\ \frac{2\nu^{k}/{\left(2-\nu \right)}^{k}+\nu^{k}\times 2\nu /\left(2-\nu \right)+\nu }{1+\left(1-2\nu^{k}/{\left(2-\nu \right)}^{k}+\nu^{k}\right)\left(1-2\nu /\left(2-\nu \right)+\nu \right)},\\ \left.\frac{2\gamma^{k}/{\left(2-\gamma \right)}^{k}+\gamma^{k}\times 2\gamma /\left(2-\gamma \right)+\gamma }{1+\left(1-2\gamma^{k}/{\left(2-\gamma \right)}^{k}+\gamma^{k}\right)\left(1-2\gamma /\left(2-\gamma \right)+\gamma \right)}\right)\\ =\left(\frac{{\left(1+\mu \right)}^{k+1}-{\left(1-\mu \right)}^{k+1}}{{\left(1+\mu \right)}^{k+1}+{\left(1-\mu \right)}^{k+1}},\frac{2\nu^{k+1}}{{\left(2-\nu \right)}^{k+1}+\nu^{k+1}},\frac{2\gamma^{k+1}}{{\left(2-\gamma \right)}^{k+1}+\gamma^{k+1}}\right)\\ =\left(\mathrm{k+}1\right)\cdot_{\varepsilon }\alpha \end{array}$$

That is, to say that equation (7) holds for *m=k+*1. Therefore, equation (7) holds for all positive integers. Now, we prove equation (7) holds for all positive real numbers. Let *λ* be any positive real number. Since 0 ≤ *μ*, *ν*, *γ*, ≤1 and 0 ≤ *μ*+*ν*+*γ* ≤ 1, we obtain 1 − *μ* ≥ *ν*, 1 − *μ* ≥ *γ*. Thus, we have 1 − *μ* ≥ *min*(*ν*, *γ*). We also have *ν* ≥ *min*(*ν*, *γ*) and *γ* ≥ *min*(*ν*, *γ*). Knowing that

(A.6) $$\begin{array}{c} \frac{{\left(1+\mu \right)}^{\lambda }-{\left(1-\mu \right)}^{\lambda }}{{\left(1+\mu \right)}^{\lambda }+{\left(1-\mu \right)}^{\lambda }}\leq 1-\frac{2{\left(1-\mu \right)}^{\lambda }}{{\left(1+\mu \right)}^{\lambda }+{\left(1-\mu \right)}^{\lambda }}\leq 1-\frac{2{\left(1-\mu \right)}^{\lambda }}{{\left(1+\mu \right)}^{\lambda }+{\left[\text{min}\left(\nu ,\gamma \right)\right]}^{\lambda }}\\ \frac{2\nu^{\lambda }}{{\left(2-\nu \right)}^{\lambda }+\nu^{\lambda }}\leq \frac{2\nu^{\lambda }}{{\left(1+\mu \right)}^{\lambda }+{\left[\text{min}\left(\nu ,\gamma \right)\right]}^{\lambda }}, \end{array}$$

and

(A.7) $$\begin{array}{c} \left.\frac{2\gamma^{\lambda }}{{\left(2-\gamma \right)}^{\lambda }+\gamma^{\lambda }}\right)\leq \frac{2\gamma^{\lambda }}{{\left(1+\mu \right)}^{\lambda }+{\left[\min\left(\nu ,\gamma \right)\right]}^{\lambda }}, \end{array}$$

we have

(A.8) $$\begin{array}{c} \frac{{\left(1+\mu \right)}^{\lambda }-{\left(1-\mu \right)}^{\lambda }}{{\left(1+\mu \right)}^{\lambda }+{\left(1-\mu \right)}^{\lambda }}+\frac{2\nu^{\lambda }}{{\left(2-\nu \right)}^{\lambda }+\nu^{\lambda }}+\frac{2\gamma^{\lambda }}{{\left(2-\gamma \right)}^{\lambda }+\gamma^{\lambda }}\\ \left.=\frac{{\left(1+\mu \right)}^{\lambda }+{\left(1-\mu \right)}^{\lambda }-2{\left(1-\mu \right)}^{\lambda }}{{\left(1+\mu \right)}^{\lambda }+{\left(1-\mu \right)}^{\lambda }}+\frac{2\nu^{\lambda }}{{\left(2-\nu \right)}^{\lambda }+\nu^{\lambda }}+\frac{2\gamma^{\lambda }}{{\left(2-\gamma \right)}^{\lambda }+\gamma^{\lambda }}\right)\\ \left.=1-\frac{2{\left(1-\mu \right)}^{\lambda }}{{\left(1+\mu \right)}^{\lambda }+{\left(1-\mu \right)}^{\lambda }}+\frac{2\nu^{\lambda }}{{\left(2-\nu \right)}^{\lambda }+\nu^{\lambda }}+\frac{2\gamma^{\lambda }}{{\left(2-\gamma \right)}^{\lambda }+\gamma^{\lambda }}\right)\\ \leq 1-\frac{2{\left(1-\mu \right)}^{\lambda }}{{\left(1+\mu \right)}^{\lambda }+{\left[\min\left(\nu ,\gamma \right)\right]}^{\lambda }}+\frac{2\nu^{\lambda }}{{\left(1+\mu \right)}^{\lambda }+{\left[\min\left(\nu ,\gamma \right)\right]}^{\lambda }}+\frac{2\gamma^{\lambda }}{{\left(1+\mu \right)}^{\lambda }+{\left[\min\left(\nu ,\gamma \right)\right]}^{\lambda }}\\ \leq 1-\frac{2{\left(\nu +\gamma \right)}^{\lambda }-2\nu^{\lambda }-2\gamma^{\lambda }}{{\left(1+\mu \right)}^{\lambda }+{\left[\text{min}\left(\nu ,\gamma \right)\right]}^{\lambda }}. \end{array}$$

Since

(A.9) $$\begin{array}{c} 2{\left(\nu +\gamma \right)}^{\lambda }-2\nu^{\lambda }-2\gamma^{\lambda }\\ =2\left[\left(\nu^{\lambda }+\nu^{\lambda -1}\gamma +\nu^{\lambda -2}\gamma^{2}+\cdots +\nu \gamma^{\lambda -1}+\gamma^{\lambda }\right)-\nu^{\lambda }-\gamma^{\lambda }\right]\\ =2\left(\nu^{\lambda -1}\gamma +\nu^{\lambda -2}\gamma^{2}+\cdots +\nu \gamma^{\lambda -1}\right)\geq 0, \end{array}$$

we have

(A.10) $$\begin{array}{c} 1-\frac{2{\left(\nu +\gamma \right)}^{\lambda }-2\nu^{\lambda }-2\gamma^{\lambda }}{{\left(1+\mu \right)}^{\lambda }+{\left[\min\left(\nu ,\gamma \right)\right]}^{\lambda }},\\ \leq 1-\frac{2\left(\nu^{\lambda -1}\gamma +\nu^{\lambda -2}\gamma^{2}+\cdots +\nu \gamma^{\lambda -1}\right)}{{\left(1+\mu \right)}^{\lambda }+{\left[\min\left(\nu ,\gamma \right)\right]}^{\lambda }}\leq 1. \end{array}$$

Furthermore,

(A.11) $$\begin{array}{c} \frac{{\left(1+\mu \right)}^{\lambda }-{\left(1-\mu \right)}^{\lambda }}{{\left(1+\mu \right)}^{\lambda }+{\left(1-\mu \right)}^{\lambda }}\geq 0,\\ \frac{2\nu^{\lambda }}{{\left(2-\nu \right)}^{\lambda }+\nu^{\lambda }}\geq 0,\\ \frac{2\gamma^{\lambda }}{{\left(2-\gamma \right)}^{\lambda }+\gamma^{\lambda }}\geq 0. \end{array}$$

With the above analysis, we have

(A.12) $$\begin{array}{c} 0\leq \frac{{\left(1+\mu \right)}^{\lambda }-{\left(1-\mu \right)}^{\lambda }}{{\left(1+\mu \right)}^{\lambda }+{\left(1-\mu \right)}^{\lambda }}+\frac{2\nu^{\lambda }}{{\left(2-v\right)}^{\lambda }+\nu^{\lambda }}+\frac{2\gamma^{\lambda }}{{\left(2-\gamma \right)}^{\lambda }+\gamma^{\lambda }}\leq 1. \end{array}$$

That is, to say, *α*_1_⊗_*ε*_*α*_2_ is also a PFV for any positive real number. Similar to *λ*·_*ε*_*α*, we can prove that *α*^*λ*^ is a PFV.

RETRACTED

### B. Proof of Theorem 4

Proof First, according to Theorem 3, it is clear that the aggregated value with picture fuzzy Einstein hybrid-weighted average (*PFEHWA*) operator is also a PFV. We now prove that equation (17) holds. According to the operations of PFVs defined in Definition 8, we have

(B.1) $$\begin{array}{c} \frac{\omega_{\varepsilon \left(j\right)}\lambda_{j}}{\sum_{j=1}^{n}\omega_{\varepsilon \left(j\right)}\lambda_{j}}\alpha_{j}=\left(\frac{{\left(1+\mu_{\alpha_{j}}\right)}^{\omega_{\varepsilon \left(j\right)}\lambda_{j}/\sum_{j=1}^{n}\omega_{\varepsilon \left(j\right)}\lambda_{j}}-{\left(1-\mu_{\alpha_{j}}\right)}^{\omega_{\varepsilon \left(j\right)}\lambda_{j}/\sum_{j=1}^{n}\omega_{\varepsilon \left(j\right)}\lambda_{j}}}{{\left(1+\mu_{\alpha_{j}}\right)}^{\omega_{\varepsilon \left(j\right)}\lambda_{j}/\sum_{j=1}^{n}\omega_{\varepsilon \left(j\right)}\lambda_{j}}+{\left(1-\mu_{\alpha_{j}}\right)}^{\omega_{\varepsilon \left(j\right)}\lambda_{j}/\sum_{j=1}^{n}\omega_{\varepsilon \left(j\right)}\lambda_{j}}}\right.\\ \left.\frac{2\nu_{\alpha_{j}}{}^{\omega_{\varepsilon \left(j\right)}\lambda_{j}/\sum_{j=1}^{n}\omega_{\varepsilon \left(j\right)}\lambda_{j}}}{{\left(2-\nu_{\alpha_{j}}\right)}^{\omega_{\varepsilon \left(j\right)}\lambda_{j}/\sum_{j=1}^{n}\omega_{\varepsilon \left(j\right)}\lambda_{j}}+\nu_{\alpha_{j}}{}^{\omega_{\varepsilon \left(j\right)}\lambda_{j}/\sum_{j=1}^{n}\omega_{\varepsilon \left(j\right)}\lambda_{j}}},\frac{2\gamma_{\alpha_{j}}{}^{\omega_{\varepsilon \left(j\right)}\lambda_{j}/\sum_{j=1}^{n}\omega_{\varepsilon \left(j\right)}\lambda_{j}}}{{\left(2-\nu_{\alpha_{j}}\right)}^{\omega_{\varepsilon \left(j\right)}\lambda_{j}/\sum_{j=1}^{n}\omega_{\varepsilon \left(j\right)}\lambda_{j}}+\gamma_{\alpha_{j}}{}^{\omega_{\varepsilon \left(j\right)}\lambda_{j}/\sum_{j=1}^{n}\omega_{\varepsilon \left(j\right)}\lambda_{j}}}\right), \end{array}$$

where *j*=1,2, ⋯ *n*. We prove the correctness of equation (17) with inductive method.

(1) for *n*=1, it is trivial.
(2) Suppose equation (17) holds for *n*=*k*, that is:
  (B.2) $$\begin{array}{c} {\text{PFEHWA}}_{\omega ,\lambda }\left(\alpha_{1},\alpha_{2},\cdots ,\alpha_{k}\right)=(\frac{\prod_{j=1}^{k}{\left(1+\mu_{\alpha_{j}}\right)}^{\omega_{\varepsilon \left(j\right)}\lambda /\sum_{j=1}^{n}\omega_{\varepsilon \left(j\right)}\lambda_{j}}-\prod_{j=1}^{k}{\left(1-\mu_{\alpha_{j}}\right)}^{\omega_{\varepsilon \left(j\right)}\lambda /\sum_{j=1}^{n}\omega_{\varepsilon \left(j\right)}\lambda_{j}}}{\prod_{j=1}^{k}{\left(1+\mu_{\alpha_{j}}\right)}^{\omega_{\varepsilon \left(j\right)}\lambda /\sum_{j=1}^{n}\omega_{\varepsilon \left(j\right)}\lambda_{j}}+\prod_{j=1}^{k}{\left(1-\mu_{\alpha_{j}}\right)}^{\omega_{\varepsilon \left(j\right)}\lambda /\sum_{j=1}^{n}\omega_{\varepsilon \left(j\right)}\lambda_{j}}}\\ \frac{2\prod_{j=1}^{k}\nu_{\alpha_{j}}{}^{\omega_{\varepsilon \left(j\right)}\lambda /\sum_{j=1}^{n}\omega_{\varepsilon \left(j\right)}\lambda_{j}}}{\prod_{j=1}^{k}{\left(2-\nu_{\alpha_{j}}\right)}^{\omega_{\varepsilon \left(j\right)}\lambda /\sum_{j=1}^{n}\omega_{\varepsilon \left(j\right)}\lambda_{j}}+\prod_{j=1}^{k}\nu_{\alpha_{j}}{}^{\omega_{\varepsilon \left(j\right)}\lambda /\sum_{j=1}^{n}\omega_{\varepsilon \left(j\right)}\lambda_{j}}}\\ \left.\frac{2\prod_{j=1}^{k}\gamma_{\alpha_{j}}{}^{\omega_{\varepsilon \left(j\right)}\lambda /\sum_{j=1}^{n}\omega_{\varepsilon \left(j\right)}\lambda_{j}}}{\prod_{j=1}^{k}{\left(2-\gamma_{\alpha_{j}}\right)}^{\omega_{\varepsilon \left(j\right)}\lambda /\sum_{j=1}^{n}\omega_{\varepsilon \left(j\right)}\lambda_{j}}+\prod_{j=1}^{k}\gamma_{\alpha_{j}}{}^{\omega_{\varepsilon \left(j\right)}\lambda /\sum_{j=1}^{n}\omega_{\varepsilon \left(j\right)}\lambda_{j}}}\right). \end{array}$$
(3) When *n*=*k*+ 1, according to Definition 9 and Theorem 3, we have as follows:
  (B.3) $$\begin{array}{c} PFEHWA_{\omega ,\lambda }\left(\alpha_{1},\alpha_{2},\cdots ,\alpha_{k},\alpha_{k+1}\right)\\ =\left(\frac{\prod_{j=1}^{k}{\left(1+\mu_{\alpha_{j}}\right)}^{\omega_{\varepsilon \left(j\right)}\lambda_{j}/\sum_{j=1}^{n}\omega_{\varepsilon \left(j\right)}\lambda_{j}}-\prod_{j=1}^{k}{\left(1-\mu_{\alpha_{j}}\right)}^{\omega_{\varepsilon \left(j\right)}\lambda /\sum_{j=1}^{n}\omega_{\varepsilon \left(j\right)}\lambda_{j}}}{\prod_{j=1}^{k}{\left(1+\mu_{\alpha_{j}}\right)}^{\omega_{\varepsilon \left(j\right)}\lambda_{j}/\sum_{j=1}^{n}\omega_{\varepsilon \left(j\right)}\lambda_{j}}+\prod_{j=1}^{k}{\left(1-\mu_{\alpha_{j}}\right)}^{\omega_{\varepsilon \left(j\right)}\lambda_{j}/\sum_{j=1}^{n}\omega_{\varepsilon \left(j\right)}\lambda_{j}}},\frac{2\prod_{j=1}^{k}\nu_{\alpha_{j}}{}^{\omega_{\varepsilon \left(j\right)}\lambda_{j}/\sum_{j=1}^{n}\omega_{\varepsilon \left(j\right)}\lambda_{j}}}{\prod_{j=1}^{k}{\left(2-\nu_{\alpha_{j}}\right)}^{\omega_{\varepsilon \left(j\right)}\lambda_{j}/\sum_{j=1}^{n}\omega_{\varepsilon \left(j\right)}\lambda_{j}}+\prod_{j=1}^{k}\nu_{\alpha_{j}}{}^{\omega_{\varepsilon \left(j\right)}\lambda_{j}/\sum_{j=1}^{n}\omega_{\varepsilon \left(j\right)}\lambda_{j}}},\right.\\ \left.\frac{2\prod_{j=1}^{k}\gamma_{\alpha_{j}}{}^{\omega_{\varepsilon \left(j\right)}\lambda_{j}/\sum_{j=1}^{n}\omega_{\varepsilon \left(j\right)}\lambda_{j}}}{\prod_{j=1}^{k}{\left(2-\gamma_{\alpha_{j}}\right)}^{\omega_{\varepsilon \left(j\right)}\lambda_{j}/\sum_{j=1}^{n}\omega_{\varepsilon \left(j\right)}\lambda_{j}}+\prod_{j=1}^{k}\gamma_{\alpha_{j}}{}^{\omega_{\varepsilon \left(j\right)}\lambda_{j}/\sum_{j=1}^{n}\omega_{\varepsilon \left(j\right)}\lambda_{j}}}\right)\\ =\left(\frac{{\left(1+\mu_{\alpha_{k+1}}\right)}^{\omega_{\varepsilon \left(k+1\right)}\lambda_{k+1}/\sum_{j=1}^{k+1}\omega_{\varepsilon \left(k+1\right)}\lambda_{k+1}}-{\left(1-\mu_{\alpha_{k+1}}\right)}^{\omega_{\varepsilon \left(k+1\right)}\lambda_{k+1}/\sum_{j=1}^{k+1}\omega_{\varepsilon \left(k+1\right)}\lambda_{k+1}}}{{\left(1+\mu_{\alpha_{k+1}}\right)}^{\omega_{\varepsilon \left(k+1\right)}\lambda_{k+1}/\sum_{j=1}^{k+1}\omega_{\varepsilon \left(k+1\right)}\lambda_{k+1}}+{\left(1-\mu_{\alpha_{k+1}}\right)}^{\omega_{\varepsilon \left(k+1\right)}\lambda_{k+1}/\sum_{j=1}^{k+1}\omega_{\varepsilon \left(k+1\right)}\lambda_{k+1}}},\frac{2\nu_{\alpha_{k+1}}{}^{\omega_{\varepsilon \left(k+1\right)}\lambda_{k+1}/\sum_{j=1}^{k+1}\omega_{\varepsilon \left(k+1\right)}\lambda_{k+1}}}{{\left(2-\nu_{\alpha_{k+1}}\right)}^{\omega_{\varepsilon \left(k+1\right)}\lambda_{k+1}/\sum_{j=1}^{k+1}\omega_{\varepsilon \left(k+1\right)}\lambda_{k+1}}+\nu_{\alpha_{k+1}}{}^{\omega_{\varepsilon \left(k+1\right)}\lambda_{k+1}/\sum_{j=1}^{k+1}\omega_{\varepsilon \left(k+1\right)}\lambda_{k+1}}},\frac{2\gamma_{\alpha_{k+1}}{}^{\omega_{\varepsilon \left(k+1\right)}\lambda_{k+1}/\sum_{j=1}^{k+1}\omega_{\varepsilon \left(k+1\right)}\lambda_{k+1}}}{{\left(2-\gamma_{\alpha_{k+1}}\right)}^{\omega_{\varepsilon \left(k+1\right)}\lambda_{k+1}/\sum_{j=1}^{k+1}\omega_{\varepsilon \left(k+1\right)}\lambda_{k+1}}+\gamma_{\alpha_{k+1}}{}^{\omega_{\varepsilon \left(k+1\right)}\lambda_{k+1}/\sum_{j=1}^{k+1}\omega_{\varepsilon \left(k+1\right)}\lambda_{k+1}}}\right)\\ =\left(\frac{\prod_{j=1}^{k}{\left(1+\mu_{\alpha_{j}}\right)}^{\omega_{\varepsilon \left(j\right)}\lambda_{j}/\sum_{j=1}^{n}\omega_{\varepsilon \left(j\right)}\lambda_{j}}-\prod_{j=1}^{k}{\left(1-\mu_{\alpha_{j}}\right)}^{\omega_{\varepsilon \left(j\right)}\lambda_{j}/\sum_{j=1}^{n}\omega_{\varepsilon \left(j\right)}\lambda_{j}}/\prod_{j=1}^{k}{\left(1+\mu_{\alpha_{j}}\right)}^{\omega_{\varepsilon \left(j\right)}\lambda_{j}/\sum_{j=1}^{n}\omega_{\varepsilon \left(j\right)}\lambda_{j}}+\prod_{j=1}^{k}{\left(1-\mu_{\alpha_{j}}\right)}^{\omega_{\varepsilon \left(j\right)}\lambda_{j}/\sum_{j=1}^{n}\omega_{\varepsilon \left(j\right)}\lambda_{j}}+{\left(1+\mu_{\alpha_{k+1}}\right)}^{\omega_{\varepsilon \left(k+1\right)}\lambda_{k+1}/\sum_{j=1}^{k+1}\omega_{\varepsilon \left(k+1\right)}\lambda_{k+1}}-{\left(1-\mu_{\alpha_{k+1}}\right)}^{\omega_{\varepsilon \left(k+1\right)}\lambda_{k+1}/\sum_{j=1}^{k+1}\omega_{\varepsilon \left(k+1\right)}\lambda_{k+1}}/{\left(1+\mu_{\alpha_{k+1}}\right)}^{\omega_{\varepsilon \left(k+1\right)}\lambda_{k+1}/\sum_{j=1}^{k+1}\omega_{\varepsilon \left(k+1\right)}\lambda_{k+1}}+{\left(1-\mu \right)}_{\alpha_{k+1}}{}^{\omega_{\varepsilon \left(k+1\right)}\lambda_{k+1}/\sum_{j=1}^{k+1}\omega_{\varepsilon \left(k+1\right)}\lambda_{k+1}}}{1+\prod_{j=1}^{k}{\left(1+\mu_{\alpha_{j}}\right)}^{\omega_{\varepsilon \left(j\right)}\lambda_{j}/\sum_{j=1}^{n}\omega_{\varepsilon \left(j\right)}\lambda_{j}}+\prod_{j=1}^{k}{\left(1-\mu_{\alpha_{j}}\right)}^{\omega_{\varepsilon \left(j\right)}\lambda_{j}/\sum_{j=1}^{n}\omega_{\varepsilon \left(j\right)}\lambda_{j}}/\prod_{j=1}^{k}{\left(1+\mu_{\alpha_{j}}\right)}^{\omega_{\varepsilon \left(j\right)}\lambda_{j}/\sum_{j=1}^{n}\omega_{\varepsilon \left(j\right)}\lambda_{j}}+\prod_{j=1}^{k}{\left(1-\mu_{\alpha_{j}}\right)}^{\omega_{\varepsilon \left(j\right)}\lambda_{j}/\sum_{j=1}^{n}\omega_{\varepsilon \left(j\right)}\lambda_{j}}\times {\left(1+\mu_{\alpha_{k+1}}\right)}^{\omega_{\varepsilon \left(k+1\right)}\lambda_{k+1}/\sum_{j=1}^{k+1}\omega_{\varepsilon \left(k+1\right)}\lambda_{k+1}}-{\left(1-\mu_{\alpha_{k+1}}\right)}^{\omega_{\varepsilon \left(k+1\right)}\lambda_{k+1}/\sum_{j=1}^{k+1}\omega_{\varepsilon \left(k+1\right)}\lambda_{k+1}}/{\left(1+\mu_{\alpha_{k+1}}\right)}^{\omega_{\varepsilon \left(k+1\right)}\lambda_{k+1}/\sum_{j=1}^{k+1}\omega_{\varepsilon \left(k+1\right)}\lambda_{k+1}}+{\left(1-\mu_{\alpha_{k+1}}\right)}^{\omega_{\varepsilon \left(k+1\right)}\lambda_{k+1}/\sum_{j=1}^{k+1}\omega_{\varepsilon \left(k+1\right)}\lambda_{k+1}}}\right.,\\ \frac{2\times 2\prod_{j=1}^{k}\nu_{\alpha_{j}}{}^{\omega_{\varepsilon \left(j\right)}\lambda_{j}/\sum_{j=1}^{n}\omega_{\varepsilon \left(j\right)}\lambda_{j}}/\prod_{j=1}^{k}{\left(2-\nu_{\alpha_{j}}\right)}^{\omega_{\varepsilon \left(j\right)}\lambda_{j}/\sum_{j=1}^{n}\omega_{\varepsilon \left(j\right)}\lambda_{j}}+\prod_{j=1}^{k}\nu_{\alpha_{j}}{}^{\omega_{\varepsilon \left(j\right)}\lambda_{j}/\sum_{j=1}^{n}\omega_{\varepsilon \left(j\right)}\lambda_{j}}\times 2\nu_{\alpha_{k+1}}{}^{\omega_{\varepsilon \left(k+1\right)}\lambda_{k+1}/\sum_{j=1}^{k+1}\omega_{\varepsilon \left(k+1\right)}\lambda_{k+1}}/{\left(2-\nu_{\alpha_{k+1}}\right)}^{\omega_{\varepsilon \left(k+1\right)}\lambda_{k+1}/\sum_{j=1}^{k+1}\omega_{\varepsilon \left(k+1\right)}\lambda_{k+1}}+\nu_{\alpha_{k+1}}{}^{\omega_{\varepsilon \left(k+1\right)}\lambda_{k+1}/\sum_{j=1}^{k+1}\omega_{\varepsilon \left(k+1\right)}\lambda_{k+1}}}{1+\left(1-2\prod_{j=1}^{k}\nu_{\alpha_{j}}{}^{\omega_{\varepsilon \left(j\right)}\lambda_{j}/\sum_{j=1}^{n}\omega_{\varepsilon \left(j\right)}\lambda_{j}}/\prod_{j=1}^{k}{\left(2-\nu_{\alpha_{j}}\right)}^{\omega_{\varepsilon \left(j\right)}\lambda_{j}/\sum_{j=1}^{n}\omega_{\varepsilon \left(j\right)}\lambda_{j}}+\prod_{j=1}^{k}\nu_{\alpha_{j}}{}^{\omega_{\varepsilon \left(j\right)}\lambda_{j}/\sum_{j=1}^{n}\omega_{\varepsilon \left(j\right)}\lambda_{j}}\right)\times \left(1-2\nu_{\alpha_{k+1}}{}^{\omega_{\varepsilon \left(k+1\right)}\lambda_{k+1}/\sum_{j=1}^{k+1}\omega_{\varepsilon \left(k+1\right)}\lambda_{k+1}}/{\left(2-\nu_{\alpha_{k+1}}\right)}^{\omega_{\varepsilon \left(k+1\right)}\lambda_{k+1}/\sum_{j=1}^{k+1}\omega_{\varepsilon \left(k+1\right)}\lambda_{k+1}}+\nu_{\alpha_{k+1}}{}^{\omega_{\varepsilon \left(k+1\right)}\lambda_{k+1}/\sum_{j=1}^{k+1}\omega_{\varepsilon \left(k+1\right)}\lambda_{k+1}}\right)}, \end{array}$$
  (B.4) $$\begin{array}{c} \frac{2\times 2\prod_{j=1}^{k}\gamma_{\alpha_{j}}{}^{\omega_{\varepsilon \left(j\right)}\lambda_{j}/\sum_{j=1}^{n}\omega_{\varepsilon \left(j\right)}\lambda_{j}}/\prod_{j=1}^{k}{\left(2-\gamma_{\alpha_{j}}\right)}^{\omega_{\varepsilon \left(j\right)}\lambda_{j}/\sum_{j=1}^{n}\omega_{\varepsilon \left(j\right)}\lambda_{j}}+\prod_{j=1}^{k}\gamma_{\alpha_{j}}{}^{\omega_{\varepsilon \left(j\right)}\lambda_{j}/\sum_{j=1}^{n}\omega_{\varepsilon \left(j\right)}\lambda_{j}}\times 2\gamma_{A_{k+1}}{}^{\omega_{\varepsilon \left(k+1\right)}\lambda_{k+1}/\sum_{j=1}^{k+1}\omega_{\varepsilon \left(k+1\right)}\lambda_{k+1}}/{\left(2-\gamma_{A_{k+1}}\right)}^{\omega_{\varepsilon \left(k+1\right)}\lambda_{k+1}/\sum_{j=1}^{k+1}\omega_{\varepsilon \left(k+1\right)}\lambda_{k+1}}+\gamma_{A_{k+1}}{}^{\omega_{\varepsilon \left(k+1\right)}\lambda_{k+1}/\sum_{j=1}^{k+1}\omega_{\varepsilon \left(k+1\right)}\lambda_{k+1}}}{1+\left(1-2\prod_{j=1}^{k}\gamma_{\alpha_{j}}{}^{\omega_{\varepsilon \left(j\right)}\lambda_{j}/\sum_{j=1}^{n}\omega_{\varepsilon \left(j\right)}\lambda_{j}}/\prod_{j=1}^{k}{\left(2-\gamma_{\alpha_{j}}\right)}^{\omega_{\varepsilon \left(j\right)}\lambda_{j}/\sum_{j=1}^{n}\omega_{\varepsilon \left(j\right)}\lambda_{j}}+\prod_{j=1}^{k}\gamma_{\alpha_{j}}{}^{\omega_{\varepsilon \left(j\right)}\lambda_{j}/\sum_{j=1}^{n}\omega_{\varepsilon \left(j\right)}\lambda_{j}}\right)\times \left(1-2\gamma_{\alpha_{k+1}}{}^{\omega_{\varepsilon \left(k+1\right)}\lambda_{k+1}/\sum_{j=1}^{k+1}\omega_{\varepsilon \left(k+1\right)}\lambda_{k+1}}/{\left(2-\gamma_{\alpha_{k+1}}\right)}^{\omega_{\varepsilon \left(k+1\right)}\lambda_{k+1}/\sum_{j=1}^{k+1}\omega_{\varepsilon \left(k+1\right)}\lambda_{k+1}}+\gamma_{\alpha_{k+1}}{}^{\omega_{\varepsilon \left(k+1\right)}\lambda_{k+1}/\sum_{j=1}^{k+1}\omega_{\varepsilon \left(k+1\right)}\lambda_{k+1}}\right)},\\ =\left(\frac{\prod_{j=1}^{k}{\left(1+\mu_{\alpha_{j}}\right)}^{\omega_{\varepsilon \left(j\right)}\lambda_{j}/\sum_{j=1}^{n}\omega_{\varepsilon \left(j\right)}\lambda_{j}}\times {\left(1+\mu_{A_{k+1}}\right)}^{\omega_{\varepsilon \left(j\right)}\lambda_{j}/\sum_{j=1}^{n}\omega_{\varepsilon \left(j\right)}\lambda_{j}}-\prod_{j=1}^{k}{\left(1-\mu_{\alpha_{j}}\right)}^{\omega_{\varepsilon \left(j\right)}\lambda /\sum_{j=1}^{n}\omega_{\varepsilon \left(j\right)}\lambda_{j}}\times {\left(1-\mu_{\alpha_{k+1}}\right)}^{\omega_{\varepsilon \left(k+1\right)}\lambda_{k+1}/\sum_{j=1}^{k+1}\omega_{\varepsilon \left(k+1\right)}\lambda_{k+1}}}{\prod_{j=1}^{k}{\left(1+\mu_{\alpha_{j}}\right)}^{\omega_{\varepsilon \left(j\right)}\lambda_{j}/\sum_{j=1}^{n}\omega_{\varepsilon \left(j\right)}\lambda_{j}}\times {\left(1+\mu_{A_{k+1}}\right)}^{\omega_{\varepsilon \left(j\right)}\lambda_{j}/\sum_{j=1}^{n}\omega_{\varepsilon \left(j\right)}\lambda_{j}}+\prod_{j=1}^{k}{\left(1-\mu_{\alpha_{j}}\right)}^{\omega_{\varepsilon \left(j\right)}\lambda_{j}/\sum_{j=1}^{n}\omega_{\varepsilon \left(j\right)}\lambda_{j}}\times {\left(1-\mu_{\alpha_{k+1}}\right)}^{\omega_{\varepsilon \left(k+1\right)}\lambda_{k+1}/\sum_{j=1}^{k+1}\omega_{\varepsilon \left(k+1\right)}\lambda_{k+1}}}\right),\\ \frac{2\prod_{j=1}^{k+1}\nu_{\alpha_{j}}{}^{\omega_{\varepsilon \left(j\right)}\lambda_{j}/\sum_{j=1}^{n}\omega_{\varepsilon \left(j\right)}\lambda_{j}}}{\prod_{j=1}^{k+1}{\left(2-\nu_{\alpha_{j}}\right)}^{\omega_{\varepsilon \left(j\right)}\lambda_{j}/\sum_{j=1}^{n}\omega_{\varepsilon \left(j\right)}\lambda_{j}}+\prod_{j=1}^{k+1}\nu_{\alpha_{j}}{}^{\omega_{\varepsilon \left(j\right)}\lambda_{j}/\sum_{j=1}^{n}\omega_{\varepsilon \left(j\right)}\lambda_{j}}},\frac{2\prod_{j=1}^{k+1}\gamma_{\alpha_{j}}{}^{\omega_{\varepsilon \left(j\right)}\lambda_{j}/\sum_{j=1}^{n}\omega_{\varepsilon \left(j\right)}\lambda_{j}}}{\prod_{j=1}^{k+1}{\left(2-\gamma_{\alpha_{j}}\right)}^{\omega_{\varepsilon \left(j\right)}\lambda_{j}/\sum_{j=1}^{n}\omega_{\varepsilon \left(j\right)}\lambda_{j}}+\prod_{j=1}^{k+1}\gamma_{\alpha_{j}}{}^{\omega_{\varepsilon \left(j\right)}\lambda_{j}/\sum_{j=1}^{n}\omega_{\varepsilon \left(j\right)}\lambda_{j}}},\\ =\left(\frac{\prod_{j=1}^{k+1}{\left(1+\mu_{\alpha_{j}}\right)}^{\omega_{\varepsilon \left(j\right)}\lambda_{j}/\sum_{j=1}^{n}\omega_{\varepsilon \left(j\right)}\lambda_{j}}-\prod_{j=1}^{k+1}{\left(1-\mu_{\alpha_{j}}\right)}^{\omega_{\varepsilon \left(j\right)}\lambda_{j}/\sum_{j=1}^{n}\omega_{\varepsilon \left(j\right)}\lambda_{j}}}{\prod_{j=1}^{k+1}{\left(1+\mu_{\alpha_{j}}\right)}^{\omega_{\varepsilon \left(j\right)}\lambda_{j}/\sum_{j=1}^{n}\omega_{\varepsilon \left(j\right)}\lambda_{j}}+\prod_{j=1}^{k+1}{\left(1-\mu_{\alpha_{j}}\right)}^{\omega_{\varepsilon \left(j\right)}\lambda_{j}/\sum_{j=1}^{n}\omega_{\varepsilon \left(j\right)}\lambda_{j}}},\frac{2\prod_{j=1}^{k+1}\nu_{\alpha_{j}}{}^{\omega_{\varepsilon \left(j\right)}\lambda_{j}/\sum_{j=1}^{n}\omega_{\varepsilon \left(j\right)}\lambda_{j}}}{\prod_{j=1}^{k+1}{\left(2-\nu_{\alpha_{j}}\right)}^{\omega_{\varepsilon \left(j\right)}\lambda_{j}/\sum_{j=1}^{n}\omega_{\varepsilon \left(j\right)}\lambda_{j}}+\prod_{j=1}^{k+1}\nu_{\alpha_{j}}{}^{\omega_{\varepsilon \left(j\right)}\lambda_{j}/\sum_{j=1}^{n}\omega_{\varepsilon \left(j\right)}\lambda_{j}}},\frac{2\prod_{j=1}^{k+1}\gamma_{A_{j}}{}^{\omega_{\varepsilon \left(j\right)}\lambda_{j}/\sum_{j=1}^{n}\omega_{\varepsilon \left(j\right)}\lambda_{j}}}{\prod_{j=1}^{k+1}{\left(2-\gamma_{\alpha_{j}}\right)}^{\omega_{\varepsilon \left(j\right)}\lambda_{j}/\sum_{j=1}^{n}\omega_{\varepsilon \left(j\right)}\lambda_{j}}+\prod_{j=1}^{k+1}\gamma_{A_{j}}{}^{\omega_{\varepsilon \left(j\right)}\lambda_{j}/\sum_{j=1}^{n}\omega_{\varepsilon \left(j\right)}\lambda_{j}}}\right) \end{array}$$

i.e., equation (17) holds for *n* = *k* + 1. That is, equation (17) holds for all *n*. So, we complete the proof of Theorem 5.

RETRACTED

### C. Proof of Theorem 5

Proof (1) Idempotency. According to Definition 4 and Theorem 3, we have

(C.1) $$\begin{array}{c} PFEHWA_{\omega ,\lambda }\left(A_{1},A_{2},\cdots ,A_{m}\right)\\ =PFEHWA_{\omega ,\lambda }\left(A,A,\cdots ,A\right)\\ =\left(\frac{\prod_{j=1}^{m}{\left(1+\mu_{A}\right)}^{\omega_{\varepsilon \left(j\right)}\lambda_{j}/\sum_{j=1}^{n}\omega_{\varepsilon \left(j\right)}\lambda_{j}}-\prod_{j=1}^{m}{\left(1-\mu_{A}\right)}^{\omega_{\varepsilon \left(j\right)}\lambda_{j}/\sum_{j=1}^{n}\omega_{\varepsilon \left(j\right)}\lambda_{j}}}{\prod_{j=1}^{m}{\left(1+\mu_{A_{j}}\right)}^{\omega_{\varepsilon \left(j\right)}\lambda_{j}/\sum_{j=1}^{n}\omega_{\varepsilon \left(j\right)}\lambda_{j}}+\prod_{j=1}^{m}{\left(1-\mu_{A_{j}}\right)}^{\omega_{\varepsilon \left(j\right)}\lambda_{j}/\sum_{j=1}^{n}\omega_{\varepsilon \left(j\right)}\lambda_{j}}},\frac{2\prod_{j=1}^{m}\nu_{A}{}^{\omega_{\varepsilon \left(j\right)}\lambda_{j}/\sum_{j=1}^{n}\omega_{\varepsilon \left(j\right)}\lambda_{j}}}{\prod_{j=1}^{m}{\left(2-\nu_{A}\right)}^{\omega_{\varepsilon \left(j\right)}\lambda_{j}/\sum_{j=1}^{n}\omega_{\varepsilon \left(j\right)}\lambda_{j}}+\prod_{j=1}^{m}\nu_{A}{}^{\omega_{\varepsilon \left(j\right)}\lambda_{j}/\sum_{j=1}^{n}\omega_{\varepsilon \left(j\right)}\lambda_{j}}},\frac{2\prod_{j=1}^{m}\gamma_{A}{}^{\omega_{\varepsilon \left(j\right)}\lambda_{j}/\sum_{j=1}^{n}\omega_{\varepsilon \left(j\right)}\lambda_{j}}}{\prod_{j=1}^{m}{\left(2-\gamma_{A}\right)}^{\omega_{\varepsilon \left(j\right)}\lambda_{j}/\sum_{j=1}^{n}\omega_{\varepsilon \left(j\right)}\lambda_{j}}+\prod_{j=1}^{m}\gamma_{A}{}^{\omega_{\varepsilon \left(j\right)}\lambda_{j}/\sum_{j=1}^{n}\omega_{\varepsilon \left(j\right)}\lambda_{j}}}\right)\\ =\left(\frac{{\left(1+\mu_{A}\right)}^{\sum_{j=1}^{m}\omega_{\varepsilon \left(j\right)}\lambda_{j}/\sum_{j=1}^{n}\omega_{\varepsilon \left(j\right)}\lambda_{j}}-{\left(1-\mu_{A}\right)}^{\sum_{j=1}^{m}\omega_{\varepsilon \left(j\right)}\lambda_{j}/\sum_{j=1}^{n}\omega_{\varepsilon \left(j\right)}\lambda_{j}}}{{\left(1+\mu_{A_{j}}\right)}^{\sum_{j=1}^{m}\omega_{\varepsilon \left(j\right)}\lambda_{j}/\sum_{j=1}^{n}\omega_{\varepsilon \left(j\right)}\lambda_{j}}+{\left(1-\mu_{A_{j}}\right)}^{\sum_{j=1}^{m}\omega_{\varepsilon \left(j\right)}\lambda_{j}/\sum_{j=1}^{n}\omega_{\varepsilon \left(j\right)}\lambda_{j}}},\frac{2\nu_{A}{}^{\sum_{j=1}^{m}\omega_{\varepsilon \left(j\right)}\lambda_{j}/\sum_{j=1}^{n}\omega_{\varepsilon \left(j\right)}\lambda_{j}}}{{\left(2-\nu_{A}\right)}^{\sum_{j=1}^{m}\omega_{\varepsilon \left(j\right)}\lambda_{j}/\sum_{j=1}^{n}\omega_{\varepsilon \left(j\right)}\lambda_{j}}+\nu_{A}{}^{\sum_{j=1}^{m}\omega_{\varepsilon \left(j\right)}\lambda_{j}/\sum_{j=1}^{n}\omega_{\varepsilon \left(j\right)}\lambda_{j}}},\frac{2\gamma_{A}{}^{\sum_{j=1}^{m}\omega_{\varepsilon \left(j\right)}\lambda_{j}/\sum_{j=1}^{n}\omega_{\varepsilon \left(j\right)}\lambda_{j}}}{{\left(2-\gamma_{A}\right)}^{\sum_{j=1}^{m}\omega_{\varepsilon \left(j\right)}\lambda_{j}/\sum_{j=1}^{n}\omega_{\varepsilon \left(j\right)}\lambda_{j}}+\gamma_{A}{}^{\sum_{j=1}^{m}\omega_{\varepsilon \left(j\right)}\lambda_{j}/\sum_{j=1}^{n}\omega_{\varepsilon \left(j\right)}\lambda_{j}}}\right) \end{array}$$

(2) Boundedness Let *f*(*x*) = (1 − *x*)/(1 + *x*), *x* ∈ [0, 1]. Then, *f*′(*x*) = −2/(1 + *x*)^2^ > 0 and thus, *f*(*x*) is a decreasing function. Since $\underset{j}{min}\mu_{A_{j}}\leq \mu_{A_{j}}\leq \underset{j}{max}\mu_{A_{j}}$, for all *j*, then $f\left(\underset{j}{\max}\mu_{A_{j}}\right)\leq f\left(\mu_{A_{j}}\right)\leq f\left(\underset{j}{\min}\mu_{A_{j}}\right)$. Let *α* = *ω*_*ε*(*j*)_*λ*_*j*_/∑_*j*=1_^*n*^*ω*_*ε*(*j*)_*λ*_*j*_. Therefore, we have as follows:

(C.2) $$\begin{array}{c} \frac{\left(1-\underset{j}{\max}\mu_{A_{j}}\right)}{\left(1+\underset{j}{\max}\mu_{A_{j}}\right)}\leq \frac{\left(1-\mu_{A_{j}}\right)}{\left(1+\mu_{A_{j}}\right)}\leq \frac{\left(1-\underset{j}{\min}\mu_{A_{j}}\right)}{\left(1+\underset{j}{\min}\mu_{A_{j}}\right)}. \end{array}$$

So, we can derive the following:

(C.3) $$\begin{array}{c} \frac{{\left(1-\underset{j}{\max}\mu_{A_{j}}\right)}^{\omega_{\varepsilon \left(j\right)}\lambda_{j}/\sum_{j=1}^{n}\omega_{\varepsilon \left(j\right)}\lambda_{j}}}{{\left(1+\underset{j}{\max}\mu_{A_{j}}\right)}^{\omega_{\varepsilon \left(j\right)}\lambda_{j}/\sum_{j=1}^{n}\omega_{\varepsilon \left(j\right)}\lambda_{j}}}\leq \frac{{\left(1-\mu_{A_{j}}\right)}^{\omega_{\varepsilon \left(j\right)}\lambda_{j}/\sum_{j=1}^{n}\omega_{\varepsilon \left(j\right)}\lambda_{j}}}{{\left(1+\mu_{A_{j}}\right)}^{\omega_{\varepsilon \left(j\right)}\lambda_{j}/\sum_{j=1}^{n}\omega_{\varepsilon \left(j\right)}\lambda_{j}}}\leq \frac{{\left(1-\underset{j}{\min}\mu_{A_{j}}\right)}^{\omega_{\varepsilon \left(j\right)}\lambda_{j}/\sum_{j=1}^{n}\omega_{\varepsilon \left(j\right)}\lambda_{j}}}{{\left(1+\underset{j}{\min}\mu_{A_{j}}\right)}^{\omega_{\varepsilon \left(j\right)}\lambda_{j}/\sum_{j=1}^{n}\omega_{\varepsilon \left(j\right)}\lambda_{j}}}. \end{array}$$

Thus,

(C.4) $$\begin{array}{c} \prod_{j=1}^{m}\frac{{\left(1-\underset{j}{max}\mu_{A_{j}}\right)}^{\omega_{\varepsilon \left(j\right)}\lambda_{j}/\sum_{j=1}^{n}\omega_{\varepsilon \left(j\right)}\lambda_{j}}}{{\left(1+\underset{j}{max}\mu_{A_{j}}\right)}^{\omega_{\varepsilon \left(j\right)}\lambda_{j}/\sum_{j=1}^{n}\omega_{\varepsilon \left(j\right)}\lambda_{j}}}\leq \prod_{j=1}^{m}\frac{{\left(1-\mu_{A_{j}}\right)}^{\omega_{\varepsilon \left(j\right)}\lambda_{j}/\sum_{j=1}^{m}\omega_{\varepsilon \left(j\right)}\lambda_{j}}}{{\left(1+\mu_{A_{j}}\right)}^{\omega_{\varepsilon \left(j\right)}\lambda_{j}/\sum_{j=1}^{m}\omega_{\varepsilon \left(j\right)}\lambda_{j}}}\leq \prod_{j=1}^{m}\frac{{\left(1-\underset{j}{min}\mu_{A_{j}}\right)}^{\omega_{\varepsilon \left(j\right)}\lambda_{j}/\sum_{j=1}^{m}\omega_{\varepsilon \left(j\right)}\lambda_{j}}}{{\left(1+\underset{j}{min}\mu_{A_{j}}\right)}^{\omega_{\varepsilon \left(j\right)}\lambda_{j}/\sum_{j=1}^{m}\omega_{\varepsilon \left(j\right)}\lambda_{j}}}\\ \Leftrightarrow \frac{{\left(1-\underset{j}{max}\mu_{A_{j}}\right)}^{\sum_{j=1}^{m}\left(\omega_{\varepsilon \left(j\right)}\lambda_{j}/\sum_{j=1}^{m}\omega_{\varepsilon \left(j\right)}\lambda_{j}\right)}}{{\left(1+\underset{j}{max}\mu_{A_{j}}\right)}^{\sum_{j=1}^{m}\left(\omega_{\varepsilon \left(j\right)}\lambda_{j}/\sum_{j=1}^{m}\omega_{\varepsilon \left(j\right)}\lambda_{j}\right)}}\leq \prod_{j=1}^{m}\frac{{\left(1-\mu_{A_{j}}\right)}^{\omega_{\varepsilon \left(j\right)}\lambda_{j}/\sum_{j=1}^{m}\omega_{\varepsilon \left(j\right)}\lambda_{j}}}{{\left(1+\mu_{A_{j}}\right)}^{\omega_{\varepsilon \left(j\right)}\lambda_{j}/\sum_{j=1}^{m}\omega_{\varepsilon \left(j\right)}\lambda_{j}}}\leq \frac{{\left(1-\underset{j}{min}\mu_{A_{j}}\right)}^{\sum_{j=1}^{m}\left(\omega_{\varepsilon \left(j\right)}\lambda_{j}/\sum_{j=1}^{m}\omega_{\varepsilon \left(j\right)}\lambda_{j}\right)}}{{\left(1+\underset{j}{min}\mu_{A_{j}}\right)}^{\sum_{j=1}^{m}\left(\omega_{\varepsilon \left(j\right)}\lambda_{j}/\sum_{j=1}^{m}\omega_{\varepsilon \left(j\right)}\lambda_{j}\right)}}\\ \Leftrightarrow \frac{1-\underset{j}{max}\mu_{A_{j}}}{1+\underset{j}{max}\mu_{A_{j}}}\leq \prod_{j=1}^{m}\frac{{\left(1-\mu_{A_{j}}\right)}^{\omega_{\varepsilon \left(j\right)}\lambda_{j}/\sum_{j=1}^{m}\omega_{\varepsilon \left(j\right)}\lambda_{j}}}{{\left(1+\mu_{A_{j}}\right)}^{\omega_{\varepsilon \left(j\right)}\lambda_{j}/\sum_{j=1}^{m}\omega_{\varepsilon \left(j\right)}\lambda_{j}}}\leq \frac{1-\underset{j}{min}\mu_{A_{j}}}{1+\underset{j}{min}\mu_{A_{j}}}\\ \Leftrightarrow \frac{2}{1+\underset{j}{max}\mu_{A_{j}}}\leq 1+\prod_{j=1}^{m}\frac{{\left(1-\mu_{A_{j}}\right)}^{\omega_{\varepsilon \left(j\right)}\lambda_{j}/\sum_{j=1}^{m}\omega_{\varepsilon \left(j\right)}\lambda_{j}}}{{\left(1+\mu_{A_{j}}\right)}^{\omega_{\varepsilon \left(j\right)}\lambda_{j}/\sum_{j=1}^{m}\omega_{\varepsilon \left(j\right)}\lambda_{j}}}\leq \frac{2}{1+\underset{j}{min}\mu_{A_{j}}}\\ \Leftrightarrow \frac{1+\underset{j}{min}\mu_{A_{j}}}{2}\leq \frac{1}{1+\prod_{j=1}^{m}{\left(1-\mu_{A_{j}}\right)}^{\omega_{\varepsilon \left(j\right)}\lambda_{j}/\sum_{j=1}^{m}\omega_{\varepsilon \left(j\right)}\lambda_{j}}/{\left(1+\mu_{A_{j}}\right)}^{\omega_{\varepsilon \left(j\right)}\lambda_{j}/\sum_{j=1}^{m}\omega_{\varepsilon \left(j\right)}\lambda_{j}}}\leq \frac{1+\underset{j}{max}\mu_{A_{j}}}{2}\\ \Leftrightarrow \underset{j}{min}\mu_{A_{j}}\leq \frac{2}{1+\prod_{j=1}^{m}{\left(1-\mu_{A_{j}}\right)}^{\omega_{\varepsilon \left(j\right)}\lambda_{j}/\sum_{j=1}^{m}\omega_{\varepsilon \left(j\right)}\lambda_{j}}/{\left(1+\mu_{A_{j}}\right)}^{\omega_{\varepsilon \left(j\right)}\lambda_{j}/\sum_{j=1}^{m}\omega_{\varepsilon \left(j\right)}\lambda_{j}}}-1\leq \underset{j}{max}\mu_{A_{j}}\\ =\underset{j}{min}\mu_{A_{j}}\leq \frac{2}{1+\prod_{j=1}^{m}{\left(1-\mu_{A_{j}}\right)}^{\omega_{\varepsilon \left(j\right)}\lambda_{j}/\sum_{j=1}^{m}\omega_{\varepsilon \left(j\right)}\lambda_{j}}/{\left(1+\mu_{A_{j}}\right)}^{\omega_{\varepsilon \left(j\right)}\lambda_{j}/\sum_{j=1}^{m}\omega_{\varepsilon \left(j\right)}\lambda_{j}}}-1\leq \underset{j}{max}\mu_{A_{j}}\\ \Leftrightarrow \underset{j}{\min}\mu_{A_{j}}\leq \frac{{\left(1+\mu_{A_{j}}\right)}^{\omega_{\varepsilon \left(j\right)}\lambda_{j}/\sum_{j=1}^{n}\omega_{\varepsilon \left(j\right)}\lambda_{j}}-{\left(1-\mu_{A_{j}}\right)}^{\omega_{\varepsilon \left(j\right)}\lambda_{j}/\sum_{j=1}^{n}\omega_{\varepsilon \left(j\right)}\lambda_{j}}}{{\left(1+\mu_{A_{j}}\right)}^{\omega_{\varepsilon \left(j\right)}\lambda_{j}/\sum_{j=1}^{n}\omega_{\varepsilon \left(j\right)}\lambda_{j}}+{\left(1-\mu_{A_{j}}\right)}^{\omega_{\varepsilon \left(j\right)}\lambda_{j}/\sum_{j=1}^{n}\omega_{\varepsilon \left(j\right)}\lambda_{j}}}\leq \underset{j}{\max}\mu_{A_{j}}. \end{array}$$

Let*g*(*y*) = (2 − *y*)/*y*, *y* ∈[0, 1]. Then, *f*′(*y*) = −2/*y*^2^ < 0, and thus, *g*(*y*) is a decreasing function. Since *min*_*j*_*ν*_*A*_*j*__ ≤ *ν*_*A*_*j*__ ≤ *max*_*j*_*ν*_*A*_*j*__ for all *j*, then *g*(min_*j*_*ν*_*A*_*j*__) ≤ *g*(*ν*_*A*_*j*__) ≤ *g*(max_*j*_*ν*_*A*_*j*__). Let *α* = *ω*_*ε*(*j*)_*λ*_*j*_/∑_*j*=1_^*n*^*ω*_*ε*(*j*)_*λ*_*j*_. According to equation (19), we have as follows:

(C.5) $$\begin{array}{c} \frac{{\left(2-{max}_{j}\nu_{A_{j}}\right)}^{\omega_{\varepsilon \left(j\right)}\lambda_{j}/\sum_{j=1}^{n}\omega_{\varepsilon \left(j\right)}\lambda_{j}}}{{max}_{j}\nu_{A_{j}}{}^{\omega_{\varepsilon \left(j\right)}\lambda_{j}/\sum_{j=1}^{n}\omega_{\varepsilon \left(j\right)}\lambda_{j}}}\leq \frac{{\left(2-\nu_{A_{j}}\right)}^{\omega_{\varepsilon \left(j\right)}\lambda_{j}/\sum_{j=1}^{n}\omega_{\varepsilon \left(j\right)}\lambda_{j}}}{\nu_{A_{j}}{}^{\omega_{\varepsilon \left(j\right)}\lambda_{j}/\sum_{j=1}^{n}\omega_{\varepsilon \left(j\right)}\lambda_{j}}}\leq \frac{{\left(2-{min}_{j}\nu_{A_{j}}\right)}^{\omega_{\varepsilon \left(j\right)}\lambda_{j}/\sum_{j=1}^{n}\omega_{\varepsilon \left(j\right)}\lambda_{j}}}{{min}_{j}\nu_{A_{j}}{}^{\omega_{\varepsilon \left(j\right)}\lambda_{j}/\sum_{j=1}^{n}\omega_{\varepsilon \left(j\right)}\lambda_{j}}} \end{array}$$

So, we can derive the following:

(C.6) $$\begin{array}{c} \frac{\prod_{j=1}^{m}{\left(2-\underset{j}{max}\nu_{A_{j}}\right)}^{\omega_{\varepsilon \left(j\right)}\lambda_{j}/\sum_{j=1}^{n}\omega_{\varepsilon \left(j\right)}\lambda_{j}}}{\prod_{j=1}^{m}\underset{j}{max}\nu_{A_{j}}{}^{\omega_{\varepsilon \left(j\right)}\lambda_{j}/\sum_{j=1}^{n}\omega_{\varepsilon \left(j\right)}\lambda_{j}}}\leq \frac{\prod_{j=1}^{m}{\left(2-\nu_{A_{j}}\right)}^{\omega_{\varepsilon \left(j\right)}\lambda_{j}/\sum_{j=1}^{n}\omega_{\varepsilon \left(j\right)}\lambda_{j}}}{\prod_{j=1}^{m}\nu_{A_{j}}{}^{\omega_{\varepsilon \left(j\right)}\lambda_{j}/\sum_{j=1}^{n}\omega_{\varepsilon \left(j\right)}\lambda_{j}}}\leq \frac{\prod_{j=1}^{m}{\left(2-\underset{j}{min}\nu_{A_{j}}\right)}^{\omega_{\varepsilon \left(j\right)}\lambda_{j}/\sum_{j=1}^{n}\omega_{\varepsilon \left(j\right)}\lambda_{j}}}{\prod_{j=1}^{m}\underset{j}{min}\nu_{A_{j}}{}^{\omega_{\varepsilon \left(j\right)}\lambda_{j}/\sum_{j=1}^{n}\omega_{\varepsilon \left(j\right)}\lambda_{j}}}\\ \Leftrightarrow \frac{2-\underset{j}{max}\nu_{A_{j}}}{\underset{j}{max}\nu_{A_{j}}}\leq \frac{\prod_{j=1}^{m}{\left(2-\nu_{A_{j}}\right)}^{\omega_{\varepsilon \left(j\right)}\lambda_{j}/\sum_{j=1}^{n}\omega_{\varepsilon \left(j\right)}\lambda_{j}}}{\prod_{j=1}^{m}\nu_{A_{j}}{}^{\omega_{\varepsilon \left(j\right)}\lambda_{j}/\sum_{j=1}^{n}\omega_{\varepsilon \left(j\right)}\lambda_{j}}}\leq \frac{2-\underset{j}{min}\nu_{A_{j}}}{\underset{j}{min}\nu_{A_{j}}}\\ \Leftrightarrow \frac{2}{\underset{j}{max}\nu_{A_{j}}}\leq \frac{\prod_{j=1}^{m}{\left(2-\nu_{A_{j}}\right)}^{\omega_{\varepsilon \left(j\right)}\lambda_{j}/\sum_{j=1}^{n}\omega_{\varepsilon \left(j\right)}\lambda_{j}}}{\prod_{j=1}^{m}\nu_{A_{j}}{}^{\omega_{\varepsilon \left(j\right)}\lambda_{j}/\sum_{j=1}^{n}\omega_{\varepsilon \left(j\right)}\lambda_{j}}}+1\leq \frac{2}{\underset{j}{min}\nu_{A_{j}}}\\ \Leftrightarrow \underset{j}{min}\nu_{A_{j}}\leq \frac{2\prod_{j=1}^{m}\nu_{A_{j}}{}^{\omega_{\varepsilon \left(j\right)}\lambda_{j}/\sum_{j=1}^{n}\omega_{\varepsilon \left(j\right)}\lambda_{j}}}{\prod_{j=1}^{m}{\left(2-\nu_{A_{j}}\right)}^{\omega_{\varepsilon \left(j\right)}\lambda_{j}/\sum_{j=1}^{n}\omega_{\varepsilon \left(j\right)}\lambda_{j}}+\prod_{j=1}^{m}\nu_{A_{j}}{}^{\omega_{\varepsilon \left(j\right)}\lambda_{j}/\sum_{j=1}^{n}\omega_{\varepsilon \left(j\right)}\lambda_{j}}}\leq \underset{j}{max}\nu_{A_{j}}. \end{array}$$

Similarly, we have as follows:

(C.7) $$\begin{array}{c} \underset{j}{\min}\gamma_{A_{j}}\leq \frac{2\prod_{j=1}^{m}\gamma_{A_{j}}{}^{\omega_{\varepsilon \left(j\right)}\lambda_{j}/\sum_{j=1}^{n}\omega_{\varepsilon \left(j\right)}\lambda_{j}}}{\prod_{j=1}^{m}{\left(2-\gamma_{A_{j}}\right)}^{\omega_{\varepsilon \left(j\right)}\lambda_{j}/\sum_{j=1}^{n}\omega_{\varepsilon \left(j\right)}\lambda_{j}}+\prod_{j=1}^{m}\gamma_{A_{j}}{}^{\omega_{\varepsilon \left(j\right)}\lambda_{j}/\sum_{j=1}^{n}\omega_{\varepsilon \left(j\right)}\lambda_{j}}}\leq \underset{j}{\max}\gamma_{A_{j}}. \end{array}$$

According to Definition 4, we can have *A*_*min*_⊆*A*⊆*A*_*max*_. (3) Monotonicity Let *A*_*j*_^1^ = (*μ*_*A*_*j*__^1^, *ν*_*A*_*j*__^1^, *γ*_*A*_*j*__^1^) and *A*_*j*_^2^ = (*μ*_*A*_*j*__^2^, *ν*_*A*_*j*__^2^, *γ*_*A*_*j*__^2^) be two collections of PFVs, and *μ*_*A*_*j*__^1^ ≤ *μ*_*A*_*j*__^2^, *ν*_*A*_*j*__^1^ ≥ *ν*_*A*_*j*__^2^ and *γ*_*A*_*j*__^1^ ≥ *γ*_*A*_*j*__^2^. Let PFEHWA_*ω*,*λ*_(*A*_1_^1^, *A*_2_^1^, ⋯, *A*_*m*_^1^) = *A*^1^ = (*μ*_*A*^1^_, *ν*_*A*^1^_, *γ*_*A*^1^_) and PFEHWA_*ω*,*λ*_(*A*_1_^2^, *A*_2_^2^, ⋯, *A*_*m*_^2^) = *A*^2^ = (*μ*_*A*^2^_, *ν*_*A*^2^_, *γ*_*A*^2^_). Let*f*(*x*) = (1 + *x*)/(1 − *x*), *x* ∈ [0, 1], *α* ∈ [0, 1]. Thus, *f*(*x*) is an increasing function. If *μ*_*A*_*j*__^1^ ≤ *μ*_*A*_*j*__^2^ for all *j*, then *f*(*μ*_*A*_*j*__^1^) ≤ *f*(*μ*_*A*_*j*__^2^), i.e., (1+*μ*_*A*_*j*__^1^)/(1 − *μ*_*A*_*j*__^1^) ≤ (1+*μ*_*A*_*j*__^2^)/(1 − *μ*_*A*_*j*__^2^). Let *α* = *ω*_*ε*(*j*)_*λ*_*j*_/∑_*j*=1_^*m*^*ω*_*ε*(*j*)_*λ*_*j*_. Therefore, we have as follows:

(C.8) $$\begin{array}{c} \frac{{\left(1+\mu_{A_{j}}^{1}\right)}^{\omega_{\varepsilon \left(j\right)}\lambda_{j}/\sum_{j=1}^{m}\omega_{\varepsilon \left(j\right)}\lambda_{j}}}{{\left(1-\mu_{A_{j}}^{1}\right)}^{\omega_{\varepsilon \left(j\right)}\lambda_{j}/\sum_{j=1}^{m}\omega_{\varepsilon \left(j\right)}\lambda_{j}}}\leq \frac{{\left(1+\mu_{A_{j}}^{2}\right)}^{\omega_{\varepsilon \left(j\right)}\lambda_{j}/\sum_{j=1}^{m}\omega_{\varepsilon \left(j\right)}\lambda_{j}}}{{\left(1-\mu_{A_{j}}^{2}\right)}^{\omega_{\varepsilon \left(j\right)}\lambda_{j}/\sum_{j=1}^{m}\omega_{\varepsilon \left(j\right)}\lambda_{j}}}. \end{array}$$

So, we can derive the following:

(C.9) $$\begin{array}{c} \frac{\prod_{i=1}^{m}{\left(1+\mu_{A_{j}}^{1}\right)}^{\omega_{\varepsilon \left(j\right)}\lambda_{j}/\sum_{j=1}^{m}\omega_{\varepsilon \left(j\right)}\lambda_{j}}}{\prod_{i=1}^{m}{\left(1-\mu_{A_{j}}^{1}\right)}^{\omega_{\varepsilon \left(j\right)}\lambda_{j}/\sum_{j=1}^{m}\omega_{\varepsilon \left(j\right)}\lambda_{j}}}\leq \frac{\prod_{i=1}^{m}{\left(1+\mu_{A_{j}}^{2}\right)}^{\omega_{\varepsilon \left(j\right)}\lambda_{j}/\sum_{j=1}^{m}\omega_{\varepsilon \left(j\right)}\lambda_{j}}}{\prod_{i=1}^{m}{\left(1-\mu_{A_{j}}^{2}\right)}^{\omega_{\varepsilon \left(j\right)}\lambda_{j}/\sum_{j=1}^{m}\omega_{\varepsilon \left(j\right)}\lambda_{j}}}\\ \Leftrightarrow 1+\frac{\prod_{i=1}^{m}{\left(1+\mu_{A_{j}}^{1}\right)}^{\omega_{\varepsilon \left(j\right)}\lambda_{j}/\sum_{j=1}^{m}\omega_{\varepsilon \left(j\right)}\lambda_{j}}}{\prod_{i=1}^{m}{\left(1-\mu_{A_{j}}^{1}\right)}^{\omega_{\varepsilon \left(j\right)}\lambda_{j}/\sum_{j=1}^{m}\omega_{\varepsilon \left(j\right)}\lambda_{j}}}\leq 1+\frac{\prod_{i=1}^{m}{\left(1+\mu_{A_{j}}^{2}\right)}^{\omega_{\varepsilon \left(j\right)}\lambda_{j}/\sum_{j=1}^{m}\omega_{\varepsilon \left(j\right)}\lambda_{j}}}{\prod_{i=1}^{m}{\left(1-\mu_{A_{j}}^{2}\right)}^{\omega_{\varepsilon \left(j\right)}\lambda_{j}/\sum_{j=1}^{m}\omega_{\varepsilon \left(j\right)}\lambda_{j}}}\\ \Leftrightarrow \frac{2}{1+\prod_{i=1}^{m}{\left(1+\mu_{A_{j}}^{2}\right)}^{\omega_{\varepsilon \left(j\right)}\lambda_{j}/\sum_{j=1}^{m}\omega_{\varepsilon \left(j\right)}\lambda_{j}}/\prod_{i=1}^{m}{\left(1-\mu_{A_{j}}^{2}\right)}^{\omega_{\varepsilon \left(j\right)}\lambda_{j}/\sum_{j=1}^{m}\omega_{\varepsilon \left(j\right)}\lambda_{j}}}\leq \frac{2}{1+\prod_{i=1}^{m}{\left(1+\mu_{A_{j}}^{1}\right)}^{\omega_{\varepsilon \left(j\right)}\lambda_{j}/\sum_{j=1}^{m}\omega_{\varepsilon \left(j\right)}\lambda_{j}}/\prod_{i=1}^{m}{\left(1-\mu_{A_{j}}^{1}\right)}^{\omega_{\varepsilon \left(j\right)}\lambda_{j}/\sum_{j=1}^{m}\omega_{\varepsilon \left(j\right)}\lambda_{j}}}\\ \Leftrightarrow 1-\frac{2}{1+\prod_{i=1}^{m}{\left(1+\mu_{A_{j}}^{1}\right)}^{\omega_{\varepsilon \left(j\right)}\lambda_{j}/\sum_{j=1}^{m}\omega_{\varepsilon \left(j\right)}\lambda_{j}}/\prod_{i=1}^{m}{\left(1-\mu_{A_{j}}^{1}\right)}^{\omega_{\varepsilon \left(j\right)}\lambda_{j}/\sum_{j=1}^{m}\omega_{\varepsilon \left(j\right)}\lambda_{j}}}\leq 1-\frac{2}{1+\prod_{i=1}^{m}{\left(1+\mu_{A_{j}}^{2}\right)}^{\omega_{\varepsilon \left(j\right)}\lambda_{j}/\sum_{j=1}^{m}\omega_{\varepsilon \left(j\right)}\lambda_{j}}/\prod_{i=1}^{m}{\left(1-\mu_{A_{j}}^{2}\right)}^{\omega_{\varepsilon \left(j\right)}\lambda_{j}/\sum_{j=1}^{m}\omega_{\varepsilon \left(j\right)}\lambda_{j}}}\\ \Leftrightarrow \frac{\prod_{i=1}^{m}{\left(1+\mu_{A_{j}}^{1}\right)}^{\omega_{\varepsilon \left(j\right)}\lambda_{j}/\sum_{j=1}^{m}\omega_{\varepsilon \left(j\right)}\lambda_{j}}-\prod_{i=1}^{m}{\left(1-\mu_{A_{j}}^{1}\right)}^{\omega_{\varepsilon \left(j\right)}\lambda_{j}/\sum_{j=1}^{m}\omega_{\varepsilon \left(j\right)}\lambda_{j}}}{\prod_{i=1}^{m}{\left(1+\mu_{A_{j}}^{1}\right)}^{\omega_{\varepsilon \left(j\right)}\lambda_{j}/\sum_{j=1}^{m}\omega_{\varepsilon \left(j\right)}\lambda_{j}}+\prod_{i=1}^{m}{\left(1-\mu_{A_{j}}^{1}\right)}^{\omega_{\varepsilon \left(j\right)}\lambda_{j}/\sum_{j=1}^{m}\omega_{\varepsilon \left(j\right)}\lambda_{j}}}\\ \leq \frac{\prod_{i=1}^{m}{\left(1+\mu_{A_{j}}^{2}\right)}^{\omega_{\varepsilon \left(j\right)}\lambda_{j}/\sum_{j=1}^{m}\omega_{\varepsilon \left(j\right)}\lambda_{j}}-\prod_{i=1}^{m}{\left(1-\mu_{A_{j}}^{2}\right)}^{\omega_{\varepsilon \left(j\right)}\lambda_{j}/\sum_{j=1}^{m}\omega_{\varepsilon \left(j\right)}\lambda_{j}}}{\prod_{i=1}^{m}{\left(1+\mu_{A_{j}}^{2}\right)}^{\omega_{\varepsilon \left(j\right)}\lambda_{j}/\sum_{j=1}^{m}\omega_{\varepsilon \left(j\right)}\lambda_{j}}+\prod_{i=1}^{m}{\left(1-\mu_{A_{j}}^{2}\right)}^{\omega_{\varepsilon \left(j\right)}\lambda_{j}/\sum_{j=1}^{m}\omega_{\varepsilon \left(j\right)}\lambda_{j}}}\\ \Leftrightarrow \mu_{A^{1}}\leq \mu_{A^{2}}. \end{array}$$

Let*g*(*y*) = (2 − *y*)/*y*, *y* ∈ [0, 1], *α* ∈ [0, 1]. Moreover, thus *g*(*y*) is an increasing function. Since *ν*_*A*_*j*_^1^_ ≥ *ν*_*A*_*j*_^2^_ for all *j*, then *g*(*ν*_*A*_*j*_^1^_) ≤ *g*(*ν*_*A*_*j*_^2^_), i.e., (2 − *ν*_*A*_*j*_^1^_)/*ν*_*A*_*j*_^1^_ ≤ (2 − *ν*_*A*_*j*_^2^_)/*ν*_*A*_*j*_^2^_. Let *α* = *ω*_*ε*(*j*)_*λ*_*j*_/∑_*j*=1_^*n*^*ω*_*ε*(*j*)_*λ*_*j*_*ω*. According to equation (20), we have as follows:

(C.10) $$\begin{array}{c} {\left(2-\nu_{A_{j}^{1}}/\nu_{A_{j}^{1}}\right)}^{\omega_{\varepsilon \left(j\right)}\lambda_{j}/\sum_{j=1}^{m}\omega_{\varepsilon \left(j\right)}\lambda_{j}}\leq {\left(2-\nu_{A_{j}^{2}}/\nu_{A_{j}^{2}}\right)}^{\omega_{\varepsilon \left(j\right)}\lambda_{j}/\sum_{j=1}^{m}\omega_{\varepsilon \left(j\right)}\lambda_{j}}\\ \Leftrightarrow \prod_{j=1}^{m}{\left(2-\nu_{A_{j}^{1}}/\nu_{A_{j}^{1}}\right)}^{\omega_{\varepsilon \left(j\right)}\lambda_{j}/\sum_{j=1}^{m}\omega_{\varepsilon \left(j\right)}\lambda_{j}}\leq \prod_{j=1}^{m}{\left(2-\nu_{A_{j}^{2}}/\nu_{A_{j}^{2}}\right)}^{\omega_{\varepsilon \left(j\right)}\lambda_{j}/\sum_{j=1}^{m}\omega_{\varepsilon \left(j\right)}\lambda_{j}}\\ \Leftrightarrow 1+\prod_{j=1}^{m}{\left(2-\nu_{A_{j}^{1}}/\nu_{A_{j}^{1}}\right)}^{\omega_{\varepsilon \left(j\right)}\lambda_{j}/\sum_{j=1}^{m}\omega_{\varepsilon \left(j\right)}\lambda_{j}}\leq 1+\prod_{j=1}^{m}{\left(2-\nu_{A_{j}^{2}}/\nu_{A_{j}^{2}}\right)}^{\omega_{\varepsilon \left(j\right)}\lambda_{j}/\sum_{j=1}^{m}\omega_{\varepsilon \left(j\right)}\lambda_{j}}\\ \Leftrightarrow \frac{2}{1+\prod_{j=1}^{m}{\left(2-\nu_{A_{j}^{2}}/\nu_{A_{j}^{2}}\right)}^{\omega_{\varepsilon \left(j\right)}\lambda_{j}/\sum_{j=1}^{m}\omega_{\varepsilon \left(j\right)}\lambda_{j}}}\leq \frac{2}{1+\prod_{j=1}^{m}{\left(2-\nu_{A_{j}^{1}}/\nu_{A_{j}^{1}}\right)}^{\omega_{\varepsilon \left(j\right)}\lambda_{j}/\sum_{j=1}^{m}\omega_{\varepsilon \left(j\right)}\lambda_{j}}}\\ \Leftrightarrow \frac{\prod_{j=1}^{m}{\left(\nu_{A_{j}^{2}}\right)}^{\omega_{\varepsilon \left(j\right)}\lambda_{j}/\sum_{j=1}^{m}\omega_{\varepsilon \left(j\right)}\lambda_{j}}}{\prod_{j=1}^{m}{\left(2-\nu_{A_{j}^{2}}\right)}^{\omega_{\varepsilon \left(j\right)}\lambda_{j}/\sum_{j=1}^{m}\omega_{\varepsilon \left(j\right)}\lambda_{j}}+\prod_{j=1}^{m}{\left(\nu_{A_{j}^{2}}\right)}^{\omega_{\varepsilon \left(j\right)}\lambda_{j}/\sum_{j=1}^{m}\omega_{\varepsilon \left(j\right)}\lambda_{j}}}\\ \leq \frac{\prod_{j=1}^{m}{\left(\nu_{A_{j}^{1}}\right)}^{\omega_{\varepsilon \left(j\right)}\lambda_{j}/\sum_{j=1}^{m}\omega_{\varepsilon \left(j\right)}\lambda_{j}}}{\prod_{j=1}^{m}{\left(2-\nu_{A_{j}^{1}}\right)}^{\omega_{\varepsilon \left(j\right)}\lambda_{j}/\sum_{j=1}^{m}\omega_{\varepsilon \left(j\right)}\lambda_{j}}+\prod_{j=1}^{m}{\left(\nu_{A_{j}^{1}}\right)}^{\omega_{\varepsilon \left(j\right)}\lambda_{j}/\sum_{j=1}^{m}\omega_{\varepsilon \left(j\right)}\lambda_{j}}}\\ \Leftrightarrow \nu_{A_{j}^{2}}\leq \nu_{A_{j}^{1}}. \end{array}$$

Similarly, we have the following:

(C.11) $$\begin{array}{c} \frac{\prod_{j=1}^{m}{\left(\gamma_{A_{j}^{2}}\right)}^{\omega_{\varepsilon \left(j\right)}\lambda_{j}/\sum_{j=1}^{m}\omega_{\varepsilon \left(j\right)}\lambda_{j}}}{\prod_{j=1}^{m}{\left(2-\gamma_{A_{j}^{2}}\right)}^{\omega_{\varepsilon \left(j\right)}\lambda_{j}/\sum_{j=1}^{m}\omega_{\varepsilon \left(j\right)}\lambda_{j}}+\prod_{j=1}^{m}{\left(\gamma_{A_{j}^{2}}\right)}^{\omega_{\varepsilon \left(j\right)}\lambda_{j}/\sum_{j=1}^{m}\omega_{\varepsilon \left(j\right)}\lambda_{j}}}\\ \leq \frac{\prod_{j=1}^{m}{\left(\gamma_{A_{j}^{1}}\right)}^{\omega_{\varepsilon \left(j\right)}\lambda_{j}/\sum_{j=1}^{m}\omega_{\varepsilon \left(j\right)}\lambda_{j}}}{\prod_{j=1}^{m}{\left(2-\gamma_{A_{j}^{1}}\right)}^{\omega_{\varepsilon \left(j\right)}\lambda_{j}/\sum_{j=1}^{m}\omega_{\varepsilon \left(j\right)}\lambda_{j}}+\prod_{j=1}^{m}{\left(\gamma_{A_{j}^{1}}\right)}^{\omega_{\varepsilon \left(j\right)}\lambda_{j}/\sum_{j=1}^{m}\omega_{\varepsilon \left(j\right)}\lambda_{j}}}\\ \Leftrightarrow \gamma_{A_{j}^{2}}\leq \gamma_{A_{j}^{1}}. \end{array}$$

According to Definition 4, we have *A*^1^⊆*A*^2^, which completes the proof of Theorem 5.
